The article "Gaussian Perturbation Specular Reflection Learning and Golden-Sine-Mechanism-Based Elephant Herding Optimization for Global Optimization Problems" was published in 2021. Journal: Comput Intell Neurosci.

# Gaussian Perturbation Specular Reflection Learning and Golden-Sine-Mechanism-Based Elephant Herding Optimization for Global Optimization Problems

**DOI:** 10.1155/2021/9922192

**Published:** 2021-07-10

**Authors:** Yuxian Duan, Changyun Liu, Song Li, Xiangke Guo, Chunlin Yang

**Affiliations:** ^1^Air and Missile Defense College, Air Force Engineering University, Xi'an 710051, China; ^2^Graduate College, Air Force Engineering University, Xi'an 710051, China; ^3^Air Traffic Control and Navigation College, Air Force Engineering University, Xi'an 710051, China

## Abstract

Elephant herding optimization (EHO) has received widespread attention due to its few control parameters and simple operation but still suffers from slow convergence and low solution accuracy. In this paper, an improved algorithm to solve the above shortcomings, called Gaussian perturbation specular reflection learning and golden-sine-mechanism-based EHO (SRGS-EHO), is proposed. First, specular reflection learning is introduced into the algorithm to enhance the diversity and ergodicity of the initial population and improve the convergence speed. Meanwhile, Gaussian perturbation is used to further increase the diversity of the initial population. Second, the golden sine mechanism is introduced to improve the way of updating the position of the patriarch in each clan, which can make the best-positioned individual in each generation move toward the global optimum and enhance the global exploration and local exploitation ability of the algorithm. To evaluate the effectiveness of the proposed algorithm, tests are performed on 23 benchmark functions. In addition, Wilcoxon rank-sum tests and Friedman tests with 5% are invoked to compare it with other eight metaheuristic algorithms. In addition, sensitivity analysis to parameters and experiments of the different modifications are set up. To further validate the effectiveness of the enhanced algorithm, SRGS-EHO is also applied to solve two classic engineering problems with a constrained search space (pressure-vessel design problem and tension-/compression-string design problem). The results show that the algorithm can be applied to solve the problems encountered in real production.

## 1. Introduction

Many challenging problems in applied mathematics and practical engineering can be considered as the processes of optimization [1]. Optimization is the process of selecting or determining the best results from a set of limited resources [2]. In general, there exist several explicit decision variables, objective functions, and constraints in optimization problems. In the real world, however, optimization problems vary widely, from single to multiobjective, from continuous to discrete, and from constrained to unconstrained. Optimization algorithms are used to obtain the values of decision variables and optimize the objective function under a certain range of constraints and search domains. If the search domain is compared to a forest, the optimization algorithm needs to find the potential area where the prey can be found. In this way, the optimization problem can be solved easily rather than laboriously.

Optimization algorithms are divided into two categories, namely, exact algorithms and heuristic algorithms. Traditional exact algorithms (e.g., branch-and-bound algorithms and dynamic programming), although capable of giving global optima infinite time, must rely on gradient information, and the runtime of the algorithm grows proportionally to the number of variables [3]. Therefore, it is difficult to achieve good results in the face of many types of nondifferentiable, noncontinuous, and complex high-dimensional problems in the real world [4]. As research has progressed, the emergence of heuristic algorithms (local search algorithm, tabu search, simulated annealing algorithm, etc.) has provided ideas for solving complex problems. Owing to the introduction of the greedy strategy and fixed search steps, the number of iterations of the algorithm is reduced [5]. For the NP-hard problem, an approximate and accurate solution can be given. However, the drawback is that such algorithms are greedy and often fall into local optima when solving complex problems, thus narrowing the scope of its application [6]. The metaheuristic algorithm that emerged later is a higher-level heuristic strategy, with a problem-independent algorithmic framework, and provides a set of guidelines and strategies for developing heuristic algorithms. In addition, it has fewer control parameters, greater randomness, more flexibility, and simplicity, can effectively handle discrete variables, and is computationally less expensive [7]. Compared with exact methods and heuristic algorithms, metaheuristic algorithms are more applicable in solving complex optimization problems. Due to its unique advantages, metaheuristics of various versions such as continuous and binary have been developed to be suitable for solving continuous and discrete optimization problems. Under this kind of tidal current, in recent years, metaheuristic algorithms have become more popular among researchers and are widely used in various fields.

Metaheuristic algorithms can be broadly classified into three categories, namely, evolutionary algorithms, physics-based algorithms, and swarm intelligence algorithms. Evolutionary algorithms were first proposed in the early 1970s and were mainly generated by simulating the concept of evolution in nature. Inspired by Darwinian biological evolution, Goldberg and Holland [8] proposed the first evolutionary algorithm, the genetic algorithm (GA), in 1988, which provides a stochastic and efficient method to perform a global search among a large number of candidate solutions. In addition, similar algorithms also include the differential evolutionary algorithm (DE) [9], biogeography-based algorithm (BBO) [10], and evolution strategy (ES) [11]. Physics-based algorithms are modeled using physical concepts and laws to update the agents in the search space, mainly including analytical modeling based on the laws of the universe, physical/chemical rules, scientific phenomena, and other ways [12]. For example, to overcome the defects that traditional GA algorithms tend to converge prematurely and have long running time, Hsiao et al. [13] proposed the space gravitational algorithm (SGA) based on the inspiration of Einstein's theory of relativity and the laws of motion of asteroids in the universe. Then, Rashedi et al. [14] proposed the gravitational search algorithm (GSA) by analyzing the interaction between gravity in the universe, which received wide attention. It has been slightly modified in the literature [15] to be adaptable to industrial applications. Inspired by the idea of GSA, Flores et al. [16] proposed the gravitational interactions optimization (GIO) algorithm, which mainly modified the nondecreasing constant, and the global search capability and local search optimization are stronger than those of the GSA. In 2019, Faramarzi et al. [17] proposed an equilibrium optimizer (EO) by simulating the mass balance model of physics to achieve the final equilibrium state (optimal result) by continuously updating the search agents. Also common are multiverse optimization (MVO) [18], electromagnetic field optimization (EFO) [19], the artificial electric field algorithm for global optimization (AEFA) [20], and lightning search algorithm (LSA) [21]. The swarm intelligence algorithms focus on artificially reproducing the social behavior and thinking concepts of various groups of organisms within nature so that the intelligence of the swarm surpasses the sum of individual intelligence. In such algorithms, multiple search agents perform the search process together, sharing location information between them, and using different operators that depend on the metaphor of each algorithm to shift the search agents to new locations [22]. On that basis, the probability of finding the optimal solution can be increased, so that the best solution can be found with low computational complexity. For example, Shi et al. [23, 24] proposed particle swarm optimization (PSO) based on the behavior of biological groups of fish, insect swarms, and bird flocks. By simulating the local interactions between individuals and the environment, a globally optimal solution can be achieved. Notably, Liu et al. [25] extended PSO by introducing chaotic sequences. The exploration and exploitation capabilities of the algorithm were effectively balanced by introducing adaptive inertia weights. A novel algorithm, called the classic self-assembly algorithm (CSA), was proposed by Zapata et al. [26]. Using PSO as a navigation mechanism, the search agents were guided to continuously move toward the constructive region. Based on the collective foraging behavior of honeybees, Karaboga [27] proposed artificial bee colony optimization (ABC) in 2005, which is simple and practical and is now one of the most cited next-generation heuristics [28]. However, in the operation of the algorithm, there may be a stagnant state, which tends to make the population fall into a local optimum [29]. In addition, to solve the multiobjective problem under complex nonlinear constraints, Yang and Deb [30] replicated the reproductive behavior of cuckoo and proposed cuckoo search (CS). Owing to the introduction of Levy flights and Levy walks [31], the convergence performance of the algorithm is improved by capturing the behavior of instantaneously moving group members instead of the simple isotropic random wandering approach. Compared with algorithms such as PSO, the CS algorithm has fewer operating parameters, can satisfy the global convergence requirement, and has been widely used [32]. In the literature [33], a CS variant, called island-based CS with polynomial mutation (iCSPM), was proposed from the perspective of improving population diversity. The strategy of the island model and Levy flight strategy were introduced to enhance the search effectiveness of the algorithm. Furthermore, Yang and Gandomi [34] proposed the bat algorithm (BA) for the predatory behavior of bats. It aims to solve single-objective and multiobjective optimization problems in continuous domain space by simulating the echo-location approach. The slime mould algorithm (SMA) was proposed by Li et al. [35] in 2020, which was a very competitive algorithm. Precup et al. [36] provided a more understandable version of SMA and introduced it for fuzzy controller tuning, extending the application of SMA. Moreover, researchers have proposed bacterial foraging optimization (BFO) (Passino) [37], krill herd (KH) (Gandomi and Alavi) [38], the artificial plant optimization algorithm (APO) (Cui and Cai) [39], grey wolf optimizer (GWO) (Mirjalili et al.) [40], crisscross optimization algorithm (CSO) (Meng et al.) [41], whale optimization algorithm (WOA) (Mirjalili and Lewis) [42], crow search algorithm (CSA) (Askarzadeh) [43], salp swarm algorithm (SSA) (Mirjalili et al.) [44], Harris hawks optimization (HHO) (Heidari et al.) [45], sailfish optimizer (SFO) (Shadravan et al.) [46], manta ray foraging optimization algorithm (MRFO) (Zhao et al.) [47], and bald eagle search (BES) (Alsattar et al.) [48].

In 2016, Wang et al. [49] developed a novel metaheuristic algorithm named elephant herding optimization (EHO) for solving global unconstrained optimization problems by studying the herding behavior of elephants in nature. According to the living habits of elephants, the activity trajectory of each baby elephant is influenced by its maternal lineage. Therefore, in EHO, the clan updating operator is used to update the distance of individual elephants in each clan relative to the position of the maternal elephant. Since in each generation male elephants must move away from the clan activity, the separating operator is introduced to perform the separation operation. It is experimentally demonstrated [50] that, for most benchmark problems, the EHO algorithm can achieve better results compared to DE, GA, and BBO algorithms. It has thus aroused plenty of research interest owing to its fewer control parameters, easy implementation, and better global optimization capability for multipeaked problems [51]. Scholars and engineers have promoted EHO in various areas of practical engineering, including wireless sensor networks [52], bioinformatics [53], emotion recognition [54], character recognition [55], and cybersecurity [56].

From the perspective of EHO, although it is a relatively effective optimization tool, there are still some shortcomings, such as the lack of mutation mechanisms, slow convergence, and the tendency to fall into local optimality, which make the algorithm limited in practical applications. In recent years, researchers have achieved numerous results to overcome the deficiencies of EHO, and the research can be divided into three aspects. The first is to mix EHO with other algorithms or strategies to improve the performance of the algorithm. For example, Javaid et al. [57] combined EHO with the GA to develop a novel algorithm, GEHO, for smart grid scheduling, which reduces the maximum cost. Wang et al. [50] mixed EHO with three different approaches, namely, cultural-based EHO, alpha-tuning EHO, and biased initialization EHO. The three approaches were tested on benchmark functions from CEC 2016 and carried out on engineering problems such as gear trains, continuous stirred-tank reactors, and three-bar truss design. Chakraborty et al. [58] proposed the IEHO algorithm, which combines EHO with opposition-based learning (OBL) and dynamic Cauchy mutation (DCM) to accelerate the convergence and improve the performance of EHO. Second, a noise interference strategy is applied [59]. To increase the population diversity of the algorithm, noise interference has become a streamlining technique. Two of the most representative are the Levy flight (LF) and chaos strategy. Xu et al. [60] proposed a novel algorithm, LFEHO, that combines Levy flight with the EHO algorithm to overcome the defects of poor convergence performance and ease of falling into local optima in the original EHO. Tuba et al. [61] introduced two different chaotic maps into the original EHO for solving the unconstrained optimization problem and tested them on the CEC 2015 benchmark function. Third, to improve the internal structure of EHO, this part of the research focused on proposing adaptive operators and stagnation prevention mechanisms. Li et al. [62] introduced a global speed strategy based on EHO to assign travel speed to each elephant and achieved good results on CEC 2014. Ismaeel et al. [63] addressed the problem of unreasonable convergence to the origin in EHO by improving the cladistic update operator and separation operator, achieving the balance between exploration and exploitation. Li et al. [64] took an original approach by extracting the previous state information of the population to guide the subsequent search process. Six variants were generated by updating the weights using random numbers and the fitness of the previous agent. The experiment results showed that the quality of the obtained solutions was higher than that of the original algorithm.

Most of the metaheuristics should be enhanced because they do not apply to complex problems, such as intricate scheduling and planning problems, big data analysis, complicated machine learning structures, and arduous modeling and classification problems. Scholars such as Dokeroglu [28] pointed out that a more fruitful research direction for metaheuristics is to optimize the internal structure of metaheuristics rather than to propose new algorithms similar to the existing ones. These are one of the motivations why this paper attempts to strengthen a new metaheuristic algorithm instead of developing a new one. Moreover, the efficiency of a metaheuristic algorithm depends on the balance between the local exploitation ability and the global exploration ability during the iterations [65]. In this regard, exploration is to explore new search spaces that require search agents to be more diverse and traversable under the operation of operators. Exploitation is characterized by the algorithm's ability to extract solutions from explored regions that are more promising in approximating the global optimal solution. In that stage, search agents played a role in converging quickly toward the optimal solution. To promote the performance of the metaheuristic algorithm, a desirable balance must be struck between these two conflicting properties.

Like a coin having two sides, there are advantages and disadvantages in every developed metaheuristic. That is exactly why each algorithm cannot be applied to all problems. According to the no free lunch (NFL) theorem [66], all algorithms cannot be regarded as a universal optimal optimizer type. In other words, the success of an algorithm does not apply to all optimization problems while solving a specific set of problems. In addition, the NFL theorem encourages innovations to improve existing optimization algorithms to enhance their performance in use. Given the constant emergence of new optimization problems and the exponential growth in the size and complexity of real-world and engineering design problems, the development and improvement of new optimizers are inevitable. Khanduja and Bhushan [67] provided evidence in their research that hybrid metaheuristic algorithms can obtain better solutions than classical metaheuristic algorithms, which inspired us a lot. From these perspectives, the study of hybrid metaheuristic algorithms has a strong practical significance and value. Therefore, in this paper, the plan is to mix the EHO algorithm with other algorithmic mechanisms to exploit the advantages of each for collaborative search and effectively improve the optimization performance.

Aiming to effectively achieve the balance between the exploration and exploitation capabilities, a Gaussian perturbation specular reflection learning and golden sine mechanism-based elephant herding optimization for global optimization problems, called SRGS-EHO, is proposed in the present paper, the main contributions of which are summarized as follows:

- First, the poor diversity and traversal of randomly generated initial populations affect the convergence performance of an algorithm. In this paper, the specular reflection learning strategy is used to generate high-quality initial populations. Moreover, Gaussian perturbation is added for the mutation to further enhance the diversity of the initial population.
- Furthermore, to improve the global optimization capabilities, the golden sine mechanism is introduced to update the position of the clan leader in the algorithm to prevent the population from falling into the local optimum. At the same time, it is made to move toward the global optimum and obtain a balance between exploitation and exploration.
- Additionally, to fully verify the effectiveness of SRGS-EHO, 23 common benchmark functions are selected as tests; the Wilcoxon rank-sum test and Friedman test are also invoked. Compared with eight other recognized metaheuristics, the performance of SRGS-EHO in terms of accuracy, convergence, and statistics is completely evaluated. In addition, sensitivity analysis to parameters and experiments of the different modifications are conducted. The aims are to analyze the impact of different parameters and modules in the algorithm on the performance of the algorithm.
- Finally, SRGS-EHO is applied to solve two practical engineering design problems (the pressure-vessel design and tension/compression string design problems), and the results are compared with those achieved using other algorithms. Experiments are conducted to test the feasibility and applicability of the proposed algorithm for solving real-world problems.

The rest of this paper is organized as follows: in Section 2, the principle of EHO is briefly introduced. A detailed introduction to the proposed Gaussian perturbation SRGS-EHO method is given in Section 3. Experiments conducted are described in Section 4, which introduces the simulation experimental procedure and the analysis. In Section 5, the experiments and analysis of SRGS-EHO for solving practical engineering problems are represented. Finally, conclusions and future work are presented in Section 6.

## 2. Elephant Herding Optimization (EHO)

Elephants are herd-dwelling creatures, usually consisting of several clans. In each clan, the herd is headed by female elephants. Male elephants, however, undertake the tasks of defending the clan and usually operate outside the clan. In EHO, each clan contains an equal number of agents. According to the algorithm, the clan leader (patriarch) is identified as the individual with the best position. Depending on the relationship with the female elephant clan leader, the position of other agents is modified by the updating operator. Meanwhile, in each generation, there are a fixed number of male elephants set to leave the clan, and these elephants are modeled by using the separating operator. In general, the EHO algorithm is divided into the initialization operation, clan updating operation, and separating operation.

### 2.1. Initialization Operation

Assuming that there are *N* elephants in the *D*-dimensional search space, the *k*_*th*_ agent in the population can be represented as *X*_*k*_=(*x*_*k*_^1^, *x*_*k*_^2^,…, *x*_*k*_^*D*^), 1 ≤ *k* ≤ *N*. Therefore, the definition of the initialized population is shown in the following equation:

(1) $$\begin{array}{c} X_{k}^{m}\left(0\right)=l^{m}+\text{rand}*\left(u^{m}-l^{m}\right), \end{array}$$

where *m* stands for dimensions, 1 ≤ *m* ≤ *D*, and *u*^*m*^ and *l*^*m*^ are the upper and lower bounds of the *m*_th_ dimension. Then, the initial population can be expressed as *X*(0)={*X*_1_(0), *X*_2_(0),…, *X*_*k*_(0)}. Next, the entire initial population must be divided into the preset clans.

### 2.2. Clan Updating Operator

At this stage, the position of each individual elephant will be updated according to its position relationship with the patriarch, which is shown as follows:

(2) $$\begin{array}{c} x_{\text{new},ci,j}=x_{ci,j}+\alpha \times \left(x_{\text{best},ci}-x_{ci,j}\right)\times r, \end{array}$$

where *x*_new,*ci*,*j*_ indicates the updated position of the agent, *x*_*ci*,*j*_ represents the current location of the agent, and *x*_best,*ci*_ is the position of the current best agent. The scale factor *α* ∈ [0,1], *r* ∈ [0,1] is a random number. Through this operation, the diversity of the population can be enhanced. When *x*_*ci*,*j*_=*x*_best,*ci*_, the patriarch of the clan cannot be updated by equation (2). To avoid this situation, it is changed to the following equation:

(3) $$\begin{array}{c} x_{\text{new},ci,j}=\beta \times x_{\text{center},ci}. \end{array}$$

The scale factor *β* ∈ [0,1] determines the extent to which *x*_center,*ci*_ acts on *x*_new,*ci*,*j*_. *x*_center,*ci*_ is the centre of clan *ci*, which is calculated by the positions of all agents. For the position of the *d*_th_ dimension, the expression of *x*_center,*ci*_ can be given as

(4) $$\begin{array}{c} x_{\text{center},ci,d}=\frac{1}{n_{ci}}\times \sum_{j=1}^{n_{ci}}x_{ci,j,d}. \end{array}$$

Among them, *d* is the dimensionality of the agent, *D* represents the total dimensionality, 1 ≤ *d* ≤ *D*, *n*_*ci*_ represents the number of agents in clan *ci*, and *x*_*ci*,*j*,*d*_ represents the *d*_th_ dimension of the *j*_th_ agent in clan *ci*.

### 2.3. Separating Operator

In EHO, a certain number of adult male elephants will leave the clan life. The separation operator acts on the elephant with the worst fitness in each clan, which is expressed as follows:

(5) $$\begin{array}{c} x_{\text{worst},ci}=x_{\min}+\left(x_{\max}-x_{\min}+1\right)\times \text{rand}, \end{array}$$

where *x*_max_ and *x*_min_ are the upper and lower bounds of agents in the population, respectively, *x*_worst,*ci*_ denotes the worst agent in clan *ci*, and rand ∈ [0,1] represents a random distribution from 0 to 1.

## 3. Proposed Algorithm

### 3.1. Motivations

EHO was proposed in 2016 with excellent global optimization capabilities, fewer control parameters, and ease of implementation, and its performance was verified in the original paper. Nevertheless, it can be observed that the original EHO suffers from the following deficiencies. First, the initialization of the original algorithm is completed randomly, which makes it difficult to guarantee diversity and traversal. Therefore, it may make the algorithm unable to converge to the best solution while increasing the runtime. Second, in the process of iteration, the position of the patriarch is determined by the total agents in the clan, which may break the balance between global exploration and local exploitation. Meanwhile, it is easy to fall into the local optimum while dealing with complex problems. Once the population has stalled, the algorithm will converge prematurely. The clan leader, being the best-positioned agent in the clan, should have stronger exploration ability. The above issues make EHO perform poorly when dealing with more complex problems.

The efficiency of metaheuristic algorithms depends mainly on striking the right balance between the global exploration and local exploitation phases. Among them, exploration is the process of exploring new search spaces, requiring search agents to be more diverse and traversable under the operation of operators. Exploitation is characterized by the algorithm's ability to extract solutions from the explored region that are more promising in approximating the global optimal solution. Therefore, search agents are desired to converge quickly toward the optimal solution. To improve the performance of the metaheuristic algorithm, a desirable balance must be struck between these two conflicting properties. If the balance is broken, the algorithm will suffer from falling into a local optimum while failing to obtain a globally optimal solution.

To deal with these problems, improvements are made in two aspects in this paper. First, specular reflection learning is introduced to update the initialization scheme. Subsequently, Gaussian perturbation is introduced to further enhance the population diversity. Second, the golden sine mechanism is presented to modify the position of the patriarch in each generation of the clan, making it converge to the global optimum continuously, improving the convergence performance by balancing the local exploitation ability and global exploration ability. With these modifications, the aim is, on the one hand, to increase the population diversity and promote convergence efficiency and, on the other hand, to strengthen exploration and exploitation capabilities and establish a balance between the two phases.

### 3.2. Gaussian Perturbation-Based Specular Reflection Learning for Initializing Populations

In metaheuristic algorithms, the diversity of initial populations can significantly affect the convergence speed and solution accuracy of intelligent algorithms [68]. However, in EHO, the lack of a priori information about the search space tends to generate the initial population using random initialization, which imposes some limitations on the update strategy of the search agents. The reason for this is that, supposing the optimal solution appears at the opposite position of the randomly generated individuals, the direction of the population advance will deviate from the optimal solution. It has been demonstrated that solutions generated by the specular reflection learning (SRL) strategy are better than those generated using only random approaches. Therefore, in this paper, specular reflection learning for population initialization is introduced and Gaussian perturbation is added to compute the opposite values of the initial population in the search space, and a mutation operation is performed on the resulting agents. Then, the opposite individual fitness values are compared with those of the original individuals to filter out the better ones for retention.

Opposition-based learning (OBL) [69] is widely used to improve metaheuristic algorithms due to its excellent performance. In OBL, a candidate solution and its opposite position are simultaneously examined to speed up the convergence. The opposite point $\bar{x}$, which is in the range [*lb*, *ub*], is defined as follows:

(6) $$\begin{array}{c} \bar{x}=lb+ub-x. \end{array}$$

Inspired by the phenomenon of specular reflection, Zhang [70] proposed specular reflection learning (SRL). In physics, there is an obvious correspondence between incident light and reflected light, as shown in Figure 1(a). Based on this phenomenon, the current solution and the reverse solution can be modeled in the way shown in Figure 1(b). Under this circumstance, it can be deduced that there is some correspondence between a solution and one of its neighbors of the opposite solution. Supposing both solutions are examined simultaneously, a better solution can be obtained. It has been demonstrated that the solutions generated by the SRL strategy are better than OBL [71]. Therefore, in this paper, specular reflection learning is introduced for population initialization. Besides, Gaussian perturbation is added to perform various operations on the generated agents. According to the results of the fitness values, the better *N* individuals are retained to form the initial population.

Suppose a point *X*=(*a*, 0) exists on the horizontal plane, and the opposite point is *X*′=(*b*, 0), ∀*X*, *X*′∈[*X*_*l*_, *X*_*u*_]. When light is incident, the angles of incidence and reflection are *α* and *β*, respectively. *O* is the midpoint of [*X*_*l*_, *X*_*u*_], *O*=(*x*_0_, 0). According to the law of reflection, the following correspondence can be obtained:

(7) $$\begin{array}{c} \alpha =\beta ⟹\;\tan\left(\alpha \right)=\frac{x_{0}-a}{A_{0}}=\frac{b-x_{0}}{B_{0}}=\tan\left(\beta \right). \end{array}$$

When *B*_0_=*μA*_0_, equation (7) can be represented as

(8) $$\begin{array}{c} b=\mu \left(x_{0}-a\right)+x_{0}\\ =\left(\mu +1\right)x_{0}-\mu a=\left(0.5\mu +0.5\right)*\left(X_{l}+X_{u}\right)-\mu a, \end{array}$$

where *μ* is the preset scale factor, and when *μ* takes on a different value, *b* is represented as

(9) $$\begin{array}{c} b=\left\{\begin{array}{cc} b_{1}, & \mu \in \left(0,1\right),\\ 2x_{0}-a, & \mu =1,\\ b_{2}, & \mu \in \left(1,+\infty \right). \end{array}\right. \end{array}$$

It can be observed that, when *μ* changes, all values of [*X*_*l*_, *X*_*u*_] can be traversed by *b*. Therefore, it can be used to initialize the population and enhance the diversity and traversal of the initial population.

Let *X*=(*x*_1_, *x*_2_,…, *x*_*n*_) be a point in *n*-dimensional space, where *x*_*i*_ ∈ [*x*_min_, *x*_max_], *i* ∈ {1,2,…, *n*}. According to the basic specular reflection model, the opposite point in equation (6) can be defined by its components:

(10) $$\begin{array}{c} x_{pi}=\left(0.5\mu +0.5\right)*\left(x_{\min}+x_{\max}\right)-\mu x_{i}. \end{array}$$

It is worth noting that the scale factor *μ* in equation (10) is set to a random number within [0,1] for the convenience of the operation. After that, *x*_*i*_ and _*x*_^*pi*^ must be merged to form a search agent of size 2*N*, where the population is {*x*_*i*_, *x*_*pi*_}. Next, the fitness of the population must be calculated, and the *N* agents with the best fitness value are selected as the initial population.

SRL can be seen as a special case of opposition-based learning, in both the current solution and the reverse solution, in order to select a better solution that can provide more opportunities for discovering the global optimal solution. It is well known that the diversity of populations has a significant impact on metaheuristic algorithms [72]. The reason is that the increase in diversity can make it more practical for the population to explore a larger search area and therefore promote a move away from the local optimum. From this perspective, there are two aspects that constrain the increase of initial population diversity in SRL. First, the method does not adjust well in small spaces. Second, the SRL method is relatively fixed. Therefore, Gaussian perturbation is introduced in the present work to perform mutation operations after generating the reverse solution. The equation is as follows:

(11) $$\begin{array}{c} x_{mi}=x_{pi}*\left(1+k*\text{randn}\left(1\right)\right), \end{array}$$

where _*x*_^*pi*^ is the current inverse solution, _*x*_^*mi*^ is the newly generated inverse solution, *k* is the weight parameter (set to 1 in this paper), and randn(1) is the matrix that generates a matrix of 1 × 1 that conforms to a standard Gaussian distribution with mean 0 and variance 1. Then, the elite solution is selected as the initialized population in the following way:

(12) $$\begin{array}{c} x_{i}=\left\{\begin{array}{cc} x_{pi}, & f\left(x_{pi}\right)<f\left(x_{mi}\right),\\ x_{mi}, & \text{else,} \end{array}\right. \end{array}$$

where *x*_*i*_ denotes the final generated *i*_th_ initialized agent, *i* ∈ [1, *N*], and the final generated initialized population is *X*_0_=(*x*_1_, *x*_2_,…, *x*_*N*_).

### 3.3. Golden Sine Mechanism

The golden sine algorithm [73] is a novel metaheuristic algorithm proposed by Tanyildizi in 2017, the design of which was inspired by the sine function in mathematics, and its agents search the solution space to approximate the optimal solution according to the golden ratio. The sine curve is defined with a range [−1,1], a period 2*π*, and has a special correspondence with the unit circle, which is shown in Figure 2. When the value of the independent variable *x*_1_ of the sine function changes, the corresponding dependent variable *y*_1_ also changes. In other words, traversing all the values of the sine function is equivalent to searching all the points on the unit circle. By introducing the golden ratio, the search space is continuously reduced and the search is conducted in the region with more hope of producing the optimal value, so as to improve the convergence efficiency. The solution process is shown in Figure 3.

When the clan update operation is completed, the individual agent with the best fitness is screened and its position updated using the golden sine mechanism in the following equation:

(13) $$\begin{array}{c} x_{\text{new},ci}=x_{\text{new},ci}*\left|\sin\left(r_{1}\right)\right|-r_{2}*\;\sin\left(r_{1}\right)*\left|m_{1}*x_{\text{best},ci}-m_{2}*x_{\text{new},ci}\right|, \end{array}$$

where *x*_best,*ci*_ represents the global best individual, *r*_1_ is the random number between [0,2*π*], *r*_2_ is the random number between [0, *π*], and *m*_1_ and *m*_2_ are the coefficient factors obtained by the following equations:

(14) $$\begin{array}{c} m_{1}=a*\left(1-\tau \right)+b*\tau , \end{array}$$

(15) $$\begin{array}{c} m_{2}=a*\tau +b*\left(1-\tau \right), \end{array}$$

where *a* and *b* are the initial values of the golden ratio, which can be adjusted according to the actual problem. *τ* represents the golden ratio, $\tau =\left(\sqrt{5}-1\right)/2$. Next, the obtained agents must be compared with the global optimal solution, and the coefficient factors *m*_1_ and *m*_2_ must be updated according to the comparison results.

When  *f*(*x*_new,*ci*_) < *f*(*x*_best,*ci*_), the update method is as follows:

(16) $$\begin{array}{c} b=m_{2},m_{2}=m_{1},m_{1}=a*\tau +b*\left(1-\tau \right) \end{array}$$

When *f*(*x*_new,*ci*_) > *f*(*x*_best,*ci*_), the equation is expressed as

(17) $$\begin{array}{c} a=m_{1},m_{1}=m_{2},m_{2}=a*\left(1-\tau \right)+b*\tau . \end{array}$$

Supposing *m*_1_=*m*_2_, the method is denoted by

(18) $$\begin{array}{c} a=\text{rand}\left(0,\pi \right),\\ b=\text{rand}\left(0,-\pi \right),\\ m_{1}=a*\tau +b*\left(1-\tau \right),m_{2}=a*\left(1-\tau \right)+b*\tau . \end{array}$$

The strategy of determining the clan leader's position by the average position is replaced by a renewed position update strategy, which, in turn, performs exploration with a strong directionality. As a result, the agents with the best fitness value can be made to continuously approach the optimal solution, obtaining a better solution in each iteration and reaching a balance between global exploration and local exploitation.

### 3.4. The Workflow of SRGS-EHO

The pseudocode of SRGS-EHO is given in Algorithm 1. The algorithm starts from initialization based on SRL and further enhances the diversity of the population through Gaussian perturbation. Next, the golden sine mechanism is introduced to optimize the position of the patriarch in each clan. The position of agents is evaluated by comparing fitness, and then continuous iteration ensues until the maximum number of iterations is reached. The flowchart of SRGS-EHO is shown in Figure 4.

## 4. Experimental Results and Discussion

To verify the effectiveness of SRGS-EHO for solving global optimization problems, experiments are conducted on 23 benchmark functions. Simultaneously, eight other different metaheuristic algorithms are selected for comparison, namely, the aforementioned EHO [49], WOA [42], EO [17], HHO [45], CSO [41], GWO [40], SFO [46], and IEHO [58]. To make the experiment fair, each algorithm is run 30 times independently on the benchmark function to ensure its stability. To better reflect the differences in performance between algorithms, the nonparametric Friedman test [74] and Wilcoxon rank-sum test [75] are invoked for statistical testing. Furthermore, different combinations of parameters and modifications are set up to analyze the impact of each parameter and module in SRGS-EHO on the performance of the algorithm. The experimental environment is an Intel® Co®TM) i5-9300H CPU @ 2.40 GHz, with 16 GB RAM running the Windows 10 operating system and the MATLAB R2019b simulation experiment platform (MathWorks, USA). Specific details about the experiments are discussed in the following sections.

### 4.1. Benchmark Functions

Twenty-three commonly used benchmark functions are selected for testing, and their basic information is shown in Table 1. Among them, F1–F7 are single-peaked functions, which have only one global optimal solution in the defined upper and lower bounds and are usually used to detect the convergence rate and exploitation capability of the algorithm. F8–F23 are multipeaked functions, among which F8–F13 are high-dimensional multipeaked functions and F14–F23 are fixed-dimensional multipeaked functions, which have multiple local extrema in the defined domain of each self-function and can detect the ability of global exploration and avoid premature convergence of the algorithm.

### 4.2. Experimental Parameter Settings

To make the experiments more credible, the values reported in the original papers or widely used in different studies are selected as parameters for the respective algorithms, which are shown in Table 2. The parameter settings are kept consistent except for those listed in the table.

### 4.3. Scalability Analysis

Since dimensionality is also a significant factor affecting the accuracy of optimization, F1–F13 are extended from 30 to 100 dimensions to verify the solving ability of the algorithms in different dimensions. When completed, the results of each algorithm must be evaluated. To make the experiments more convincing, the evaluation indexes are chosen as the mean (Ave) and standard deviation (Std). Among them, the mean value can reflect the solution accuracy and quality of the algorithm, and Std reflects the stability of the algorithm. When solving the minimization problem, the smaller the mean value, the better the algorithm performance. Similarly, the smaller the standard deviation, the more stable the algorithm performance. In addition, the maximum number of iterations *t*_max_ for all algorithms is set to 500 and the overall size *N* is set to 30.

Table 3 shows the experimental results when *d*=30. As can be seen from the data, SRGS-EHO obtains the best solution on five of the seven single-peak functions (F1–F7). It is noteworthy that SRGS-EHO achieves a more significant advantage over the other algorithms on F1–F4. This is due to the introduction of the golden sine mechanism, which increases the local search ability of the algorithm, thus enhancing the exploitation ability as a result. In the performance of the multipeak functions (F8–F23), SRGS-EHO achieves the best results on F8–F11, F17, and F21–F23 and the best mean value on F14. All of the results obtained by SRGS-EHO are better than those obtained by the original EHO. This indicates that the algorithm has boosted its global capability compared to the original EHO after introducing SRL and updating the clan updating operator. In addition, the performance of multimodal functions with fixed dimensions shows that the algorithm strongly achieves a balance between exploitation and exploration.

Tables 4 and 5 show the results when the dimension was increased to 50 and 100, respectively. The data in the tables indicate that the difficulty in gaining optimal solutions is lifted as the size of the problem increases. It can be seen from Table 4 that SRGS-EHO achieves the optimal solutions in F1–F4 and F7–F11. When *d*=100, SRGS-EHO still achieves the best results in nine of the 13 benchmark functions. Combining the results from the two tables, it can be noted that the performance of SRGS-EHO does not degrade, proving that SRGS-EHO has good adaptability for handling high-dimensional problems. This indicates that the introduced Gaussian perturbation-based SRL can effectively enhance the population diversity. Moreover, the clan positions are updated by the golden sine mechanism to continuously approach the global optimum, which effectively balances early exploration and later exploitation.

### 4.4. Analysis of Convergence Curves

To further compare the convergence performance of various algorithms in solving optimization problems, the convergence curves of nine algorithms are plotted and shown in Figure 5. Among them, the dimensions of F1–F13 functions are set to 30. It is observed that the convergence accuracy of SRGS-EHO is more prominent on single-peaked functions (F1–F7), which is a great improvement compared with other algorithms. In the performance of multipeaked functions (F8–F23), SRGS-EHO converges to the global optimum on F8–F11, F14, F17, and F21–F23 and can maintain a better convergence rate. Compared with the original EHO, the convergence performance of SRGS-EHO has been significantly improved. The modifications for the initialized population and the strategy of introducing the golden sine mechanism are proved to be effective. The experimental results indicate that the optimization ability and convergence performance of SRGS-EHO are enhanced.

### 4.5. Statistical Tests

Garcia et al. [76] pointed out that, when evaluating the performance of metaheuristic algorithms, comparisons only based on mean and standard deviation are not sufficient. Moreover, there exist inevitable chance factors that affect the experimental results during the process of iteration [77]. Therefore, statistical tests are necessary to reflect the superiority of the proposed algorithm and the variability of other algorithms [78]. In this paper, the Wilcoxon rank-sum test and Friedman test are chosen to compare the performance between algorithms. Besides, the maximum number of iterations *t*_max_ of all algorithms is set to 500 and the overall size of the population *N*is set to 30. Other parameters are set as in Section 4.2. As usual, *f*_1_(*x*) to *f*_13_(*x*) are extended from 30 to 100 dimensions.

In the Wilcoxon rank-sum test, the significance level *p* is set to 0.05. When *p* < 0.05, the algorithm is proved to be statistically superior. The results of the experiments are shown in Tables 6 and 7. The notation “+/−/ = ” indicates that the proposed methods are superior to, equal to, or worse than the current method, respectively. Since the best algorithm on a benchmark function cannot be compared with itself, the best algorithm on each benchmark function is marked as NaN, which means “not applicable.”

The results show that when *d*=30, the proposed SRGS-EHO outperforms EHO, WOA, EO, HHO, CSO, GWO, SFO, and IEHO on 9, 11, 10, 8, 13, 10, and 11 problems out of 13 benchmark functions, while it underperforms them on 4, 2, 2, 2, 0, 0, 3, and 2 problems. When the dimensionality is expanded to 50 dimensions, the proposed SRGS-EHO performs better on 8, 11, 10, 7, 13, 9, and 10 problems and underperforms on 5, 2, 2, 3, 0, 0, 4, and 3 problems in comparison with the other 8 algorithms. When the dimensionality is further expanded to 100 dimensions, SRGS-EHO continues to perform more superior. It outperforms EHO, WOA, EO, HHO, CSO, GWO, SFO, and IEHO on 10, 11, 11, 9, 13, 9, and 10 benchmark functions, respectively. The performance on 3, 0, 1, 1, 0, 0, 4, and 3 problems is inferior. For the performance of the 10 fixed-dimensional benchmark functions F14–F23, SRGS-EHO performs better on 6, 10, 9, 9, 9, 7, 10, and 6 problems, respectively, while inferior to other algorithms on 4, 0, 1, 1, 1, 1, 0, 0, and 4 problems. The results show that the proposed SRGS-EHO is superior in terms of solution accuracy. Undoubtedly, the results are statistically significant.

To make the experiment more convincing, the Friedman test is performed to screen the difference between the proposed SRGS-EHO and other algorithms. As one of the most well-known and widely used statistical tests, the Friedman test is used to detect significant differences between the results of two or more algorithms on consecutive data [79]. Specifically, it can be used for multiple comparisons between different algorithms by calculating the ranking *F*_*c*_ of the experimental results. The equation is represented as

(19) $$\begin{array}{c} F_{c}=\frac{12N}{k\left(k+1\right)}\left[\sum_{j}R_{j}^{2}-\frac{k{\left(k+1\right)}^{2}}{4}\right], \end{array}$$

where *k* is the number of algorithms involved in the comparison, *j* is the correlation coefficient, *N* is the number of test cases or runs, and *R*_*j*_ is the average ranking of each algorithm.

The experimental results of Friedman tests are shown in Table 8. According to the results of the Friedman test, the algorithm with the lowest ranking is considered to be the most efficient algorithm. From the results in the table, the proposed SRGS-EHO is always ranked first in different cases (*d*=30,50,100). Compared with other metaheuristics, the SRGS-EHO has a greater competitive advantage.

### 4.6. Sensitivity Analysis to Parameters

To examine the effect of different parameters in SRGS-EHO on the performance of the algorithm, sensitivity analysis to parameters is also performed in this section. The initial values of the golden ratio *a* and *b* in equations (14) and (15), the maximum number of iterations *t*_max_, and the size of population *N* are set to different values to verify. In this experiment, *N* is set to 5, 20, and 50, *t*_max_ is marked as 100 and 500, and *a* and *b* are set to two different sets of values [−*π*, *π*] and [0,1]. Twelve variants of SRGS-EHO are created, each representing a combination of different parameters, as shown in Table 9. It should be noted that these parameters can be adapted to the actual problem.

When each seed algorithm is performed 30 times, the results of the Friedman test reported are shown in Table 10. The analysis of the data in the table yields that the quality of the obtained solutions varies if the set parameters are changed. By comparison, the subalgorithm SRGS-EHO6 with *N*=50, *t*_max_=500, *a*=−*π*,  and *b*=*π* outperforms the other variants and achieves the highest ranking.

### 4.7. Analysis of the Modifications

In order to analyze the impact of the newly tuned modules on the algorithm performance, comparison experiments are conducted in this section. In SRGS-EHO, the initialized populations are first generated by specular reflection learning based on Gaussian variational perturbations (SR-GM). Secondly, the golden sine operator (GSO) is introduced to optimize the positions of the patriarch. For a simple analysis, four algorithms, EHO, SR-GM + EHO, GSO + EHO, and SRGS-EHO, are considered to compare behaviors for solving different problems. The different strategies are combined in the way shown in Table 11. Six representative benchmark functions are selected, including F1, F5, F10, F14, F15, and F17. The size of the population *N* is set to 30 and the maximum number of iterations *t*_max_ is 500.

Figure 6 shows the convergence curves of the four algorithms. It can be seen that the convergence rate of SR-GM is generally higher than that of EHO due to the optimized initialization method using Gaussian perturbation-based specular reflection learning. The introduction of the golden sine operator makes GSO a very significant improvement in search accuracy and breadth. By combining the two strategies, the convergence rate and the search accuracy of SRGS-EHO are simultaneously promoted.

The mean value and Friedman ranking results obtained by different combinations of strategies are shown in Table 12, where the bold values indicate the best solutions obtained on the current benchmark functions. According to these results, all three enhanced versions outperform the original algorithm. Both SR-GM + EHO and GSO + EHO outperform EHO on five functions. On the one hand, SR-GM + EHO and GSO + EHO achieve different improvements in terms of the accuracy and breadth of the search compared to EHO. On the other hand, the performance of SRGS-EHO is enhanced comprehensively by the effective combination of SR-GM and GSO. By verification, it is shown that the modifications for EHO are effective. Meanwhile, SRGS-EHO is determined to be the final optimized version.

## 5. Applications of SRGS-EHO for Solving Engineering Problems

The applicability of SRGS-EHO is further tested in solving engineering design problems and the results are described here. In this paper, two restricted practical engineering test problems, namely, the pressure-vessel design and tension/compression string design problems, are selected, and the results obtained by SRGS-EHO are compared with other algorithms to highlight superiority.

It is noteworthy that these two cases include some inequality constraints. Consequently, constraint handling methods should be used in SRGS-EHO and other compared methods. Constraint handling methods are divided into five categories, namely, penalty function methods, hybrid methods, separation of objective function and constraints, repair algorithms, and special operators [80]. In terms of penalty functions, there exist different types, including static, annealing, adaptive, coevolutionary, and death penalty. Among these, the death penalty is a popular and simplest constraint processing method. In this approach, search agents that violate any level of constraints impose the same penalty, i.e., being assigned a poorer fitness value. This approach does not require any modification of the original algorithm. Constraints are added to the fitness function and are efficiently handled by most optimization algorithms. Therefore, in this study, SRGS-EHO is merged with the death penalty approach for solving constrained engineering problems. It is worth noting that the objective of solving real engineering problems is to provide the global optimal solution at the lowest possible cost. Based on this consideration, in this section, each compared algorithm is performed 10 times and the best combination and the maximum fitness value obtained are selected as the final comparison results.

### 5.1. Pressure-Vessel Design Problem

The pressure-vessel design problem [81] is a common engineering design problem first proposed by Kannan and Kramer in 1994, which is shown in Figure 7. The objective of this optimization problem is to minimize the manufacturing cost of the pressure vessel. Four variables are involved: the thickness of the shell *T*_*s*_, that of the head *T*_*h*_, and the inner radius *R* and length *L* of the cylinder. Among them, the first two variables are discrete. In addition, the problem contains four constraints. Of these, three constraints are linear and one constraint is nonlinear. The mathematical form of the problem is expressed as follows:

(20) $$\begin{array}{c} \min\;F_{4}\left(x\right)=0.6224x_{1}x_{3}x_{4}+1.7781x_{2}x_{3}^{2}+19.84x_{1}^{2}x_{3}+3.1661x_{1}^{2}x_{4}\\ \text{where }x=\left[x_{1},x_{2},x_{3},x_{4}\right]=\left[T_{s},T_{h},R,L\right]\\ \text{s}.\text{t}.\;g_{1}\left(x\right)=-x_{1}+0.0193x_{3}\leq 0g_{2}\left(x\right)=-x_{2}+0.00954x_{3}\leq 0\\ g_{3}\left(x\right)=-\frac{4}{3}\pi x_{3}^{3}-\pi x_{3}^{2}x_{4}+1296000\leq 0\\ g_{4}\left(x\right)=x_{4}-240\leq 0\\ 1\times 0.0625\leq x_{1},x_{2}\leq 99\times 0.0625\\ 10\leq x_{3},x_{4}\leq 200. \end{array}$$

SRGS-EHO is applied to optimize the problem and compared with eight other algorithms separately, with some as listed earlier, i.e., EO [17], WOA [42], HHO [45], DE [9], evolution strategies (ESs) [82], PSO [23], the opposition-based sine cosine algorithm (OBSCA) [83], improved sine cosine algorithm (ISCA) [22], and enhanced whale optimization algorithm (EWOA) [84]. The obtained results are shown in Table 13. According to the results, SRGS-EHO obtained the best solution among the nine algorithms. The four variables are optimized to 0.850468, 0.420387, 44.065679, and 153.694517, and the optimum cost obtained is 6020.753071.

### 5.2. Tension/Compression String Design Problem

This problem was described by Arora [85] and Belegundu [86] for the purpose of minimizing the weight of a tension/compression spring. Three variables are included in Figure 8, namely, diameter (*d*), mean coil diameter (*D*), and number of active coils (*P*). SRGS-EHO is applied to solve the problem and compared with eight other algorithms, namely, the slap swarm algorithm (SSA) [44], WOA [42], PSO [23], GA [87], moth-flame optimization (MFO) [88], GWO [40], the enhanced WOA (EWOA) [84], IEHO [89], and the reinforced variant of WOA (RDWOA) [90]. The results are presented in Table 10. The mathematical form of the tension/compression string design problem is expressed as follows:

(21) $$\begin{array}{c} \min\;F_{4}\left(x\right)=\left(x_{3}+2\right)x_{2}x_{1}^{2}\\ \text{where }x=\left[x_{1},x_{2},x_{3}\right]=\left[d,D,P\right]\\ \text{s}.\text{t}.\;g_{1}\left(x\right)=1-\frac{x_{2}^{3}x_{3}}{71785x_{1}^{4}}\leq 0\\ g_{2}\left(x\right)=\frac{4x_{2}^{2}-x_{1}x_{2}}{12566\left(x_{2}x_{1}^{3}-x_{1}^{4}\right)}+\frac{1}{5108x_{1}^{2}}-1\leq 0\\ g_{3}\left(x\right)=1-\frac{140.45x_{1}}{x_{2}^{2}x_{3}}\leq 0\\ g_{4}\left(x\right)=\frac{x_{1}+x_{2}}{1.5}-1\leq 0\\ 0.05\leq x_{1}\leq 2.00\\ 0.25\leq x_{2}\leq 1.30\\ 2.00\leq x_{3}\leq 15.0. \end{array}$$

As can be observed from Table 14, the optimum weight obtained by SRGS-EHO is 0.012044 when *d*, *D*, and *N* are optimized to 0.061414, 0.638027, and 3.004913, respectively. This indicates that SRGS-EHO has a superior global optimization capability compared to other algorithms.

## 6. Conclusions and Future Work

In this paper, the Gaussian perturbation-based specular reflection learning and golden sine mechanism are introduced for dealing with the defective problem of the original EHO. According to the method proposed in this paper, the population initialization method and the clan leader position update strategy are optimized, which makes exploration and exploitation more efficient and leads to the enhancement of the algorithm performance. Experiments on 23 benchmark functions show that the proposed SRGS-EHO has an excellent performance in terms of optimization accuracy and stability compared with other metaheuristic algorithms, while the convergence rate is also promoted. In addition, SRGS-EHO is applied to solve real-world engineering design problems, such as pressure-vessel design and tension/compression string design problems. Compared with other algorithms, this indicates that SRGS-EHO has superiority and applicability. At the same time, the algorithm has great potential for dealing with different complex problems.

In the future, SRGS-EHO can be further developed and refined based on practical problems. In addition, it can be introduced to solve discrete and multiobjective optimization problems, and more encouraging results can potentially be achieved.

## Figures and Tables

**Figure 1:** Diagram of specular reflection learning. (a) Specular reflection phenomenon. (b) Specular reflection model.

**Figure 2:** Correspondence between sine function and unit circle.

**Figure 3:** Schematic of solution of golden sine mechanism.

**Figure 4:** Flowchart of SRGS-EHO.

**Figure 5:** Convergence curves of different algorithms on 23 benchmark functions.

**Figure 6:** Convergence curves of different strategy combinations on 6 benchmark functions. (a) F1, (b) F5, (c) F10, (d) F14, (e) F15, and (f) F17.

**Figure 7:** Pressure-vessel design.

**Figure 8:** Tension/compression spring design problem.

**Algorithm 1:** SRGS-EHO.

**Table 1:** Details of 23 benchmark functions.

No.	Function	Dimension	Range	*f*_min_
F1	*f*_1_(*x*)=∑_*i*=1_^*n*^*x*_*i*_^2^*f*_2_(*x*)=∑_*i*=1_^*n*^|*x*_*i*_|+∏_*i*=1_^*n*^|*x*_*i*_|	30	[−100,100]	0
F2	*f*_2_(*x*)=∑_*f*_min__^*n*^|*x*_*i*_|+∏_*i*=1_^*n*^|*x*_*i*_|	30	[−10,10]	0
F3	*f*_3_(*x*)=∑_*i*=1_^*n*^(∑_*j*−1_^*i*^*x*_*j*_)^2^	30	[−100,100]	0
F4	$f_{4}\left(x\right)=\underset{i}{\min}\left\{\left|x_{i}\right|,1\leq i\leq n\right\}$	30	[−100,100]	0
F5	*f*_5_(*x*)=∑_*i*=1_^*n*−1^100(*x*_*i*+1_ − *x*_*i*_^2^)^2^+(*x*_*i*_ − 1)^2^	30	[−30,30]	0
F6	*f*_6_(*x*)=∑_*i*=1_^*n*^([*x*_*i*_+0.5])^2^	30	[−100,100]	0
F7	*f*_7_(*x*)=∑_*i*=1_^*n*^*ix*_*i*_^4^+random[0,1)	30	[−1.28,1.28]	0
F8	$f_{8}\left(x\right)=\sum_{i=1}^{n}-x_{i}\sin\left(\sqrt{\left|x_{i}\right|}\right)$	30	[−500,500]	$\begin{array}{c} -418.9829\\ \times \dim \end{array}$
F9	*f*_9_(*x*)=∑_*i*=1_^*n*^[*x*_*i*_^2^ − 10 cos(2*πx*_*i*_)+10]	30	[−5.12,5.12]	0
F10	$f_{10}\left(x\right)=-20\;\exp\left(-0.2\sqrt{\frac{1}{n}\sum_{i=1}^{n}x_{i}^{2}}\right)-\exp\left(\left(1/n\right)\sum_{i=1}^{n}\cos\left(2\pi x_{i}\right)\right)+20+e$	30	[−32,32]	0
F11	$f_{11}\left(x\right)=1/4000\sum_{i=1}^{n}\sum x_{i}^{2}-\prod_{i=1}^{n}\cos\left(x_{i}/\sqrt{i}\right)+1$	30	[−600,600]	0
F12	$\begin{array}{c} f_{12}\left(x\right)=\pi /n\left\{\sum_{i=1}^{n-1}{\left(y_{i}-1\right)}^{2}\left[1+10\;\sin^{2}\left(\pi y_{i+1}\right)\right]+{\left(y_{n}-1\right)}^{2}\right\}\\ +\sum_{i=1}^{n}u\left(x_{i},10,100,4\right)+\pi /n10\;\sin\left(\pi y_{1}\right)\\ y_{i}=1+x_{i}+\left(1/4\right)u\left(x_{i},a,k,m\right)=\left\{\begin{array}{cc} k{\left(x_{i}-a\right)}^{m} & x_{i}>a\\ 0 & -a<x_{i}<a\\ k{\left(-x_{i}-a\right)}^{m} & x_{i}<-a \end{array}\right. \end{array}$	30	[−50,50]	0
F13	$\begin{array}{c} f_{13}\left(x\right)=0.1\left\{\sum_{i=1}^{n}{\left(x_{i}-1\right)}^{2}\left[1+\;\sin^{2}\left(3\pi x_{i}+1\right)\right]+{\left(x_{n}-1\right)}^{2}\left[1+\;\sin^{2}\left(2\pi x_{n}\right)\right]\right\}\\ +0.1\sin^{2}\left(3\pi x_{1}\right)+\sum_{i=1}^{n}u\left(x_{i},5,100,4\right) \end{array}$	30	[−50,50]	0
F14	*f*_14_(*x*)=((1/500)+∑_*j*=1_^25^1/*j*+∑_*i*=1_^2^(*x*_*i*_ − *a*_*ij*_)^6^)^−1^	2	[−65,65]	1
F15	*f*_15_(*x*)=∑_*i*=1_^11^[*a*_*i*_ − *x*_1_(*b*_*i*_^2^+*b*_*i*_*x*_2_)/*b*_*i*_^2^+*b*_*i*_*x*_3_+*x*_4_]^2^	4	[−5,5]	0.00030
F16	*f*_16_(*x*)=4*x*_1_^2^ − 2.1*x*_1_^4^+1/3*x*_1_^6^+*x*_1_*x*_2_ − 4*x*_2_^2^+4*x*_2_^4^	2	[−5,5]	−1.0316
F17	*f*_17_(*x*)=(*x*_2_ − 5.1/4*π*^2^*x*_1_^2^+5/*πx*_1_ − 6)^2^+10(1 − (1/8*π*))cos *x*_1_+10	2	[−5,5]	0.398
F18	$\begin{array}{c} f_{18}\left(x\right)=\left[1+{\left(x_{1}+x_{2}+1\right)}^{2}\left(19-14x_{1}+3x_{1}^{2}-14x_{2}+6x_{1}x_{2}+3x_{2}^{2}\right)\right]\times \\ \left[30+{\left(2x_{1}-3x_{2}\right)}^{2}\times \left(18-32x_{1}+12x_{1}^{2}+48x_{2}-36x_{1}x_{2}+27x_{2}^{2}\right)\right] \end{array}$	2	[−2,2]	3
F19	*f*_19_(*x*)=−∑_*i*=1_^4^*c*_*i*_exp[−∑_*j*=1_^3^*a*_*ij*_(*x*_*j*_ − *p*_*ij*_)^2^]	3	[1, 3]	−3.86
F20	*f*_20_(*x*)=−∑_*i*=1_^4^*c*_*i*_exp[−∑_*j*=1_^6^*a*_*ij*_(*x*_*j*_ − *p*_*ij*_)^2^]	6	[0,1]	−3.32
F21	*f*_21_(*x*)=−∑_*i*=1_^5^[(*X* − *a*_*i*_)(*X* − *a*_*i*_)^*T*^+*c*_*i*_]^−1^	4	[0,10]	−10.1532
F22	*f*_22_(*x*)=−∑_*i*=1_^7^[(*X* − *a*_*i*_)(*X* − *a*_*i*_)^*T*^+*c*_*i*_]^−1^	4	[0,10]	−10.4028
F23	*f*_23_(*x*)=−∑_*i*=1_^10^[(*X* − *a*_*i*_)(*X* − *a*_*i*_)^*T*^+*c*_*i*_]^−1^	4	[0,10]	−10.5363

**Table 2:** Parameter settings of different algorithms.

Algorithm	Parameter	Range
Elephant herding optimization (EHO)	*α*	0.5
	*β*	0.1
	*N*	5
	*n*_*j*_	7

Whale optimization algorithm (WOA)	*a*	Decreased from 2 to 0
	*a*_2_	Decreased from 2 to 1
	*b*	1

Equilibrium optimizer (EO)	*a*_1_	2
	*a*_2_	1
	GP	0.5

Harris hawk optimization (HHO)	*β*	1.5
	*E*_0_	[−1,1]

Crisscross optimization algorithm (CSO)	*c*_1_	[−1,1]
	*c*_2_	[−1,1]

Grey wolf optimizer (GWO)	*a*	Decreased from 2 to 0
	*A*	4

Sailed fish optimizer (SFO)	*e*	0.001
	Initial population for the sailfish	9
	Initial population for the sardine	21

Improved elephant herding optimization (IEHO)	*α*	0.5
	*β*	0.1
	*N*	5
	*n*_*j*_	7

**Table 3:** Comparison results of 23 benchmark functions (*d*=30).

Function		SRGS-EHO	EHO	WOA	EO	HHO	CSO	GWO	SFO	IEHO
F1	Mean	**1.73E** − **268**	6.63*E* − 05	8.47*E* − 75	2.17*E* − 41	2.32*E* − 94	1.98*E* − 09	2.11*E* − 27	8.36*E* − 11	1.06*E* − 04
	Std	**0.00E** + **00**	1.46*E* − 04	3.49*E* − 74	4.68*E* − 41	1.25*E* − 93	4.41*E* − 09	3.23*E* − 27	1.78*E* − 10	2.55*E* − 04

F2	Mean	**4.88E** − **134**	4.04*E* − 03	1.55*E* − 50	6.19*E* − 24	1.33*E* − 50	3.02*E* − 07	8.75*E* − 17	4.18*E* − 05	3.70*E* − 03
	Std	**2.67E** − **133**	5.13*E* − 03	6.56*E* − 50	5.96*E* − 24	5.77*E* − 50	2.42*E* − 07	5.79*E* − 17	3.61*E* − 05	3.22*E* − 03

F3	Mean	**4.05E** − **257**	3.98*E* − 02	4.83*E* + 04	7.30*E* − 09	9.22*E* − 69	1.43*E* + 03	9.27*E* − 05	1.61*E* − 08	1.97*E* − 02
	Std	**0.00E** + **00**	8.32*E* − 02	1.56*E* + 04	2.53*E* − 08	5.05*E* − 68	7.91*E* + 02	4.40*E* − 04	1.90*E* − 08	4.29*E* − 02

F4	Mean	**7.42E** − **125**	1.08*E* − 03	4.45*E* + 01	1.42*E* − 10	9.72*E* − 50	9.79*E* − 01	5.29*E* − 07	1.44*E* − 06	1.18*E* − 03
	Std	**4.06E** − **124**	1.18*E* − 03	2.64*E* + 01	1.59*E* − 10	3.20*E* − 49	5.03*E* − 01	4.31*E* − 07	1.73*E* − 06	1.28*E* − 03

F5	Mean	1.27*E* + 00	2.77*E* − 01	2.81*E* + 01	2.53*E* + 01	**9.95E** − **03**	8.97*E* + 01	2.70*E* + 01	2.85*E* − 02	1.15*E* − 01
	Std	3.22*E* + 00	8.89*E* − 01	4.71*E* − 01	1.91*E* − 01	**1.11E** − **02**	1.93*E* + 02	8.48*E* − 01	3.03*E* − 02	1.61*E* − 01

F6	Mean	6.99*E* − 01	1.65*E* − 03	4.74*E* − 01	**8.90E** − **06**	7.80*E* − 05	9.47*E* − 10	7.20*E* − 01	3.38*E* − 02	2.20*E* − 03
	Std	1.83*E* + 00	3.61*E* − 03	2.43*E* − 01	**5.38E** − **06**	1.27*E* − 04	2.26*E* − 09	3.31*E* − 01	1.26*E* − 01	3.68*E* − 03

F7	Mean	**7.40E** − **05**	1.39*E* − 03	3.39*E* − 03	9.70*E* − 04	1.27*E* − 04	3.21*E* − 03	1.98*E* − 03	3.87*E* − 04	1.69*E* − 03
	Std	**8.74E** − **05**	1.45*E* − 03	4.00*E* − 03	4.55*E* − 04	1.23*E* − 04	2.76*E* − 03	9.00*E* − 04	3.08*E* − 04	2.16*E* − 03

F8	Mean	−**1.26E** + **04**	−1.26*E* + 04	−1.05*E* + 04	−8.94*E* + 03	−1.25*E* + 04	−1.17*E* + 04	−6.40*E* + 03	−3.83*E* + 03	−1.26*E* + 04
	Std	**2.05E** − **01**	9.84*E* + 00	1.78*E* + 03	6.59*E* + 02	3.76*E* + 02	4.83*E* + 02	1.01*E* + 03	4.04*E* + 02	1.85*E* + 01

F9	Mean	**0.00E** + **00**	6.72*E* − 05	3.79*E* − 15	**0.00E** + **00**	**0.00E** + **00**	3.40*E* − 03	3.85*E* + 00	7.31*E* − 07	5.11*E* − 05
	Std	**0.00E** + **00**	9.93*E* − 05	2.08*E* − 14	**0.00E** + **00**	**0.00E** + **00**	1.53*E* − 02	5.16*E* + 00	1.94*E* − 06	1.22*E* − 04

F10	Mean	**8.88E** − **16**	2.16*E* − 03	3.73*E* − 15	8.47*E* − 15	**8.88E** − **16**	7.19*E* − 06	1.03*E* − 13	4.23*E* − 06	1.95*E* − 03
	Std	**0.00E** + **00**	2.61*E* − 03	2.70*E* − 15	1.80*E* − 15	**0.00E** + **00**	8.89*E* − 06	2.05*E* − 14	4.04*E* − 06	2.64*E* − 03

F11	Mean	**0.00E** + **00**	1.37*E* − 04	1.17*E* − 02	9.02*E* − 04	**0.00E** + **00**	1.94*E* − 01	7.24*E* − 03	3.38*E* − 12	1.64*E* − 04
	Std	**0.00E** + **00**	2.39*E* − 04	4.45*E* − 02	4.94*E* − 03	**0.00E** + **00**	2.72*E* − 01	1.28*E* − 02	4.87*E* − 12	4.51*E* − 04

F12	Mean	8.29*E* − 09	2.77*E* − 05	5.69*E* − 02	5.74*E* − 07	5.27*E* − 06	**6.43E** − **11**	4.60*E* − 02	8.74*E* − 03	3.97*E* − 05
	Std	2.24*E* − 08	4.04*E* − 05	1.09*E* − 01	4.49*E* − 07	5.65*E* − 06	**2.46E** − **10**	2.00*E* − 02	2.22*E* − 02	7.42*E* − 05

F13	Mean	6.81*E* − 07	3.66*E* − 04	5.08*E* − 01	2.94*E* − 02	1.42*E* − 04	**1.23E** − **10**	6.25*E* − 01	7.19*E* − 05	6.70*E* − 04
	Std	2.22*E* − 06	4.42*E* − 04	2.16*E* − 01	5.94*E* − 02	1.63*E* − 04	**1.68E** − **10**	2.59*E* − 01	5.05*E* − 05	1.10*E* − 03

F14	Mean	**9.98E** − **01**	9.98*E* − 01	3.84*E* + 00	9.98*E* − 01	1.39*E* + 00	2.23*E* + 00	4.49*E* + 00	7.76*E* + 00	9.98*E* − 01
	Std	1.02*E* − 03	2.08*E* − 04	4.03*E* + 00	**1.75E** − **16**	9.56*E* − 01	2.79*E* + 00	4.08*E* + 00	3.48*E* + 00	7.26*E* − 05

F15	Mean	1.64*E* − 04	1.58*E* − 03	1.22*E* − 03	1.08*E* − 03	3.96*E* − 04	1.55*E* − 03	3.09*E* − 03	**3.55*E*** − **04**	1.66*E* − 03
	Std	1.28*E* − 04	2.75*E* − 04	3.33*E* − 03	3.65*E* − 03	2.48*E* − 04	3.28*E* − 03	6.90*E* − 03	**3.66*E*** − **05**	3.44*E* − 04

F16	Mean	−7.47*E* − 01	−7.33*E* − 01	−**1.03E** + **00**	−1.03*E* + 00	−1.03*E* + 00	−1.03*E* + 00	−1.03*E* + 00	−1.03*E* + 00	−6.73*E* − 01
	Std	4.27*E* − 01	3.70*E* − 01	**2.86E** − **09**	6.45*E* − 16	3.10*E* − 09	1.12*E* − 02	2.40*E* − 08	3.80*E* − 03	4.28*E* − 01

F17	Mean	**3.98E** − **01**	5.27*E* − 01	3.98*E* − 01	3.98*E* − 01	3.98*E* − 01	4.26*E* − 01	3.98*E* − 01	3.99*E* − 01	5.37*E* − 01
	Std	**6.54E** − **06**	2.00*E* − 01	7.71*E* − 06	4.83*E* − 05	4.04*E* − 05	8.96*E* − 02	6.39*E* − 04	1.03*E* − 03	1.78*E* − 01

F18	Mean	1.60*E* + 01	2.65*E* + 01	3.00*E* + 00	**3.00E** + **00**	3.00*E* + 00	4.73*E* + 00	3.00*E* + 00	7.73*E* + 00	1.83*E* + 01
	Std	1.00*E* + 01	8.84*E* + 00	2.52*E* − 04	**1.55E** − **15**	4.59*E* − 07	6.38*E* + 00	3.65*E* − 05	7.82*E* + 00	1.03*E* + 01

F19	Mean	−3.85*E* + 00	−3.47*E* + 00	−3.86*E* + 00	−**3.86E** + **00**	−3.86*E* + 00	−3.85*E* + 00	−3.86*E* + 00	−3.84*E* + 00	−3.49*E* + 00
	Std	2.16*E* − 06	2.44*E* − 01	6.43*E* − 03	**2.45E** − **15**	3.15*E* − 03	2.49*E* − 02	1.34*E* − 03	2.28*E* − 02	2.94*E* − 01

F20	Mean	−2.24*E* + 00	−1.89*E* + 00	−3.24*E* + 00	−3.26*E* + 00	−3.10*E* + 00	−**3.26*E*** + **00**	−3.25*E* + 00	−2.92*E* + 00	−2.24*E* + 00
	Std	4.57*E* − 01	5.59*E* − 01	1.19*E* − 01	6.70*E* − 02	1.19*E* − 01	**5.63*E*** − **02**	8.02*E* − 02	2.12*E* − 01	3.75*E* − 01

F21	Mean	−**1.01E** + **01**	−1.01*E* + 01	−8.43*E* + 00	−8.97*E* + 00	−5.21*E* + 00	−8.98*E* + 00	−9.31*E* + 00	−1.01*E* + 01	−1.01*E* + 01
	Std	**1.65E** − **02**	2.76*E* − 02	2.43*E* + 00	2.46*E* + 00	8.81*E* − 01	2.44*E* + 00	1.92*E* + 00	8.99*E* − 02	2.71*E* − 02

F22	Mean	−**1.04E** + **01**	−1.04*E* + 01	−7.64*E* + 00	−9.79*E* + 00	−5.43*E* + 00	−9.32*E* + 00	−1.02*E* + 01	−1.02*E* + 01	−1.04*E* + 01
	Std	**1.11E** − **02**	2.21*E* − 02	2.92*E* + 00	1.89*E* + 00	1.32*E* + 00	2.50*E* + 00	9.70*E* − 01	2.49*E* − 01	1.40*E* − 02

F23	Mean	−**1.05E** + **01**	−1.05*E* + 01	−6.57*E* + 00	−9.45*E* + 00	−5.13*E* + 00	−9.05*E* + 00	−1.05*E* + 01	−1.04*E* + 01	−1.05*E* + 01
	Std	**6.54E** − **06**	2.67*E* − 02	3.39*E* + 00	2.52*E* + 00	1.20*E* + 00	3.03*E* + 00	8.85*E* − 04	1.62*E* − 01	3.24*E* − 02

**Table 4:** Comparison results of 13 benchmark functions (*d*=50).

Function		SRGS-EHO	EHO	WOA	EO	HHO	CSO	GWO	SFO	IEHO
F1	Mean	**9.11E **−** 258**	2.48*E* − 04	1.95*E* − 69	1.33*E* − 34	1.42*E* − 95	5.96*E* − 04	9.71*E* − 20	1.43*E* − 10	2.37*E* − 04
	Std	**0.00E** + **00**	4.10*E* − 04	1.06*E* − 68	1.93*E* − 34	5.49*E* − 95	1.54*E* − 03	1.21*E* − 19	2.38*E* − 10	4.45*E* − 04

F2	Mean	**1.15E **−** 124**	4.05*E* − 03	7.59*E* − 50	1.54*E* − 20	1.50*E* − 50	1.47*E* − 03	2.67*E* − 12	6.00*E* − 05	1.13*E* − 02
	Std	**6.32E **−** 124**	3.93*E* − 03	3.10*E* − 49	1.57*E* − 20	6.49*E* − 50	3.73*E* − 04	1.43*E* − 12	5.78*E* − 05	1.29*E* − 02

F3	Mean	**3.91E **−** 261**	6.72*E* − 02	1.98*E* + 05	4.90*E* − 04	9.04*E* − 72	6.75*E* + 03	1.93*E* − 01	7.41*E* − 08	1.58*E* − 01
	Std	**0.00E** + **00**	1.15*E* − 01	5.13*E* + 04	9.56*E* − 04	4.58*E* − 71	2.98*E* + 03	3.53*E* − 01	1.04*E* − 07	2.37*E* − 01

F4	Mean	**7.85E **−** 134**	1.10*E* − 03	6.84*E* + 01	3.79*E* − 07	3.44*E* − 47	5.92*E* + 00	5.16*E* − 04	1.26*E* − 06	1.64*E* − 03
	Std	**3.72E **−** 133**	1.14*E* − 03	2.61*E* + 01	5.97*E* − 07	1.73*E* − 46	1.65*E* + 00	4.48*E* − 04	1.04*E* − 06	2.42*E* − 03

F5	Mean	2.79 *E* + 00	2.89*E* − 01	4.83*E* + 01	4.60*E* + 01	**3.18E **−** 02**	1.30*E* + 02	4.75*E* + 01	5.54*E* − 02	1.91*E* − 01
	Std	6.98 *E* + 00	6.62*E* − 01	3.70*E* − 01	8.85*E* − 01	**5.28E **−** 02**	6.72*E* + 01	8.83*E* − 01	8.38*E* − 02	4.35*E* − 01

F6	Mean	6.42*E* − 01	2.63*E* − 03	1.26*E* + 00	3.89*E* − 02	2.66*E* − 04	**2.58E **−** 04**	2.80*E* + 00	2.43*E* − 02	1.46*E* − 03
	Std	2.35 *E* + 00	7.36*E* − 03	5.01*E* − 01	8.59*E* − 02	4.51*E* − 04	**1.81E **−** 04**	7.33*E* − 01	7.15*E* − 02	1.97*E* − 03

F7	Mean	**6.27E **−** 05**	1.69*E* − 03	3.77*E* − 03	1.78*E* − 03	1.50*E* − 04	1.13*E* − 02	3.65*E* − 03	6.09*E* − 04	2.06*E* − 03
	Std	**5.79E **−** 05**	2.34*E* − 03	3.79*E* − 03	6.59*E* − 04	1.57*E* − 04	5.78*E* − 03	1.55*E* − 03	5.35*E* − 04	2.41*E* − 03

F8	Mean	−**2.09E** + **04**	−2.09*E* + 04	−1.69*E* + 04	−1.44*E* + 04	−2.09*E* + 04	−1.88*E* + 04	−9.13*E* + 03	−4.94*E* + 03	−2.09*E* + 04
	Std	**2.76E** + **00**	8.46*E* + 00	3.35*E* + 03	9.97*E* + 02	1.90*E* + 00	7.31*E* + 02	8.56*E* + 02	4.60*E* + 02	4.33*E* + 00

F9	Mean	**0.00E** + **00**	1.14*E* − 04	1.89*E* − 15	**0.00E** + **00**	**0.00E** + **00**	4.46*E* + 00	4.15*E* + 00	5.36*E* − 07	1.37*E* − 04
	Std	**0.00E** + **00**	2.00*E* − 04	1.04*E* − 14	**0.00E** + **00**	**0.00E** + **00**	2.95*E* + 00	5.93*E* + 00	1.21*E* − 06	2.18*E* − 04

F10	Mean	**8.88E **−** 16**	1.95*E* − 03	3.97*E* − 15	1.57*E* − 14	**8.88E **−** 16**	2.86*E* − 03	4.10*E* − 11	5.68*E* − 06	2.97*E* − 03
	Std	**0.00E** + **00**	3.84*E* − 03	2.76*E* − 15	2.96*E* − 15	**0.00E** + **00**	1.55*E* − 03	2.45*E* − 11	7.25*E* − 06	3.62*E* − 03

F11	Mean	**0.00E** + **00**	1.17*E* − 04	7.33*E* − 03	**0.00E** + **00**	**0.00E** + **00**	2.12*E* − 01	4.31*E* − 03	3.78*E* − 12	3.07*E* − 04
	Std	**0.00E** + **00**	3.43*E* − 04	4.02*E* − 02	**0.00E** + **00**	**0.00E** + **00**	3.10*E* − 01	8.60*E* − 03	7.52*E* − 12	7.04*E* − 04

F12	Mean	8.94*E* − 06	3.25*E* − 05	2.65*E* − 02	2.83*E* − 03	8.85*E* − 06	**1.12E **−** 06**	1.07*E* − 01	1.71*E* − 02	2.53*E* − 05
	Std	1.86*E* − 05	6.24*E* − 05	1.50*E* − 02	1.14*E* − 02	1.42*E* − 05	**1.10E **−** 06**	4.05*E *** **−** **02	5.35*E *** **−** **02	5.19*E *** **−** **05

F13	Mean	7.92*E *** **−** **03	2.95*E *** **−** **04	1.12*E* + 00	4.83*E *** **−** **01	7.44*E *** **−** **05	7.80*E *** **−** **05	2.10*E* + 00	**7.03E **−** 05**	1.75*E *** **−** **03
	Std	2.53*E *** **−** **02	3.92*E *** **−** **04	4.66*E *** **−** **01	2.40*E *** **−** **01	1.00*E *** **−** **04	1.59*E *** **−** **04	2.87*E *** **−** **01	**6.56E **−** 05**	3.36*E *** **−** **03

**Table 5:** Comparison results of 13 benchmark functions (*d*=100).

Function		SRGS-EHO	EHO	WOA	EO	HHO	CSO	GWO	SFO	IEHO
F1	Mean	**8.01E **−** 272**	3.23*E *** **−** **04	3.22*E *** **−** **74	3.51*E *** **−** **29	6.15*E *** **−** **94	3.98*E* + 00	1.73*E *** **−** **12	3.34*E *** **−** **10	3.29*E *** **−** **04
	Std	**0.00E** + **00**	4.55*E *** **−** **04	1.11*E *** **−** **73	4.42*E *** **−** **29	2.89*E *** **−** **93	1.60*E* + 00	1.25*E *** **−** **12	5.44*E *** **−** **10	8.21*E *** **−** **04

F2	Mean	**1.02E **−** 134**	1.26*E *** **−** **02	1.23*E *** **−** **49	2.21*E *** **−** **17	1.31*E *** **−** **48	6.58*E *** **−** **01	4.34*E *** **−** **08	1.18*E *** **−** **04	1.58*E *** **−** **02
	Std	**4.58E **−** 134**	1.98*E *** **−** **02	5.65*E *** **−** **49	3.19*E *** **−** **17	5.55*E *** **−** **48	1.07*E *** **−** **01	1.65*E *** **−** **08	1.33*E *** **−** **04	1.16*E *** **−** **02

F3	Mean	**3.34E **−** 250**	1.37*E* + 00	1.09*E* + 06	6.74*E* + 00	3.73*E *** **−** **58	3.21*E* + 04	5.53*E* + 02	2.48*E *** **−** **06	1.16*E* + 00
	Std	**0.00E** + **00**	2.47*E* + 00	3.08*E* + 05	1.53*E* + 01	1.90*E *** **−** **57	9.70*E* + 03	4.84*E* + 02	6.36*E *** **−** **06	1.65*E* + 00

F4	Mean	**8.88E **−** 133**	1.70*E *** **−** **03	7.37*E* + 01	3.88*E *** **−** **03	3.06*E *** **−** **48	1.77*E* + 01	6.85*E *** **−** **01	1.58*E *** **−** **06	1.37*E *** **−** **03
	Std	**4.85E **−** 132**	5.40*E *** **−** **03	2.54*E* + 01	9.63*E *** **−** **03	1.57*E *** **−** **47	2.71*E* + 00	7.43*E *** **−** **01	1.44*E *** **−** **06	1.67*E *** **−** **03

F5	Mean	3.69*E* + 00	9.01*E *** **−** **01	9.82*E* + 01	9.67*E* + 01	**3.40E **−** 02**	8.12*E* + 02	9.80*E* + 01	5.79*E *** **−** **02	3.51*E *** **−** **01
	Std	1.78*E *** **−** **01	1.56*E* + 00	1.70*E *** **−** **01	1.05*E* + 00	4.68*E *** **−** **02	**2.60E** + **02**	5.16*E *** **−** **01	5.90*E *** **−** **02	1.05*E* + 00

F6	Mean	3.08*E* + 00	3.80*E *** **−** **03	4.25*E* + 00	3.75*E* + 00	**3.06E **−** 04**	3.50*E* + 00	9.89*E* + 00	1.61*E *** **−** **01	4.90*E *** **−** **03
	Std	6.64*E* + 00	6.58*E *** **−** **03	1.49*E* + 00	6.54*E *** **−** **01	**5.20E **−** 04**	1.43*E* + 00	9.98*E *** **−** **01	4.87*E *** **−** **01	9.87*E *** **−** **03

F7	Mean	**8.80E **−** 05**	1.78*E *** **−** **03	5.33*E *** **−** **03	2.61*E *** **−** **03	1.16*E *** **−** **04	1.06*E *** **−** **01	5.88*E *** **−** **03	5.07*E *** **−** **04	1.98*E *** **−** **03
	Std	**1.06E **−** 04**	2.97*E *** **−** **03	6.58*E *** **−** **03	8.76*E *** **−** **04	1.18*E *** **−** **04	2.88*E *** **−** **02	2.19*E *** **−** **03	3.89*E *** **−** **04	2.85*E *** **−** **03

F8	Mean	−**4.19E** + **04**	−4.19*E* + 04	−3.52*E* + 04	−2.55*E* + 04	−4.17*E* + 04	−3.39*E* + 04	−1.63*E* + 04	−6.85*E* + 03	−4.19*E* + 04
	Std	**5.21E** + **00**	2.16*E* + 01	5.73*E* + 03	1.99*E* + 03	1.14*E* + 03	1.92*E* + 03	1.19*E* + 03	6.50*E* + 02	2.60*E* + 01

F9	Mean	**0.00E** + **00**	2.73*E *** **−** **03	**0.00E** + **00**	**0.00E** + **00**	**0.00E** + **00**	4.44*E* + 01	9.52*E* + 00	3.59*E *** **−** **07	8.80*E *** **−** **04
	Std	**0.00E** + **00**	1.34*E *** **−** **02	**0.00E** + **00**	**0.00E** + **00**	**0.00E** + **00**	9.23*E* + 00	6.45*E* + 00	5.06*E *** **−** **07	2.41*E *** **−** **03

F10	Mean	**8.88E **−** 16**	1.70*E *** **−** **03	4.20*E *** **−** **15	3.57*E *** **−** **14	**8.88E **−** 16**	7.01*E *** **−** **01	1.31*E *** **−** **07	4.56*E *** **−** **06	2.13*E *** **−** **03
	Std	**0.00E** + **00**	2.24*E *** **−** **03	2.79*E *** **−** **15	5.31*E *** **−** **15	**0.00E** + **00**	3.61*E *** **−** **01	4.74*E *** **−** **08	5.54*E *** **−** **06	2.19*E *** **−** **03

F11	Mean	**0.00E** + **00**	2.45*E *** **−** **04	8.45*E *** **−** **03	5.77*E *** **−** **04	**0.00E** + **00**	9.21*E *** **−** **01	4.21*E *** **−** **03	1.12*E *** **−** **11	1.02*E *** **−** **03
	Std	**0.00E** + **00**	2.96*E *** **−** **04	4.63*E *** **−** **02	3.16*E *** **−** **03	**0.00E** + **00**	1.21*E *** **−** **01	9.79*E *** **−** **03	1.63*E *** **−** **11	2.45*E *** **−** **03

F12	Mean	2.21*E *** **−** **05	1.47*E *** **−** **04	4.67*E *** **−** **02	4.15*E *** **−** **02	**3.48E **−** 06**	4.38*E *** **−** **02	3.17*E *** **−** **01	1.44*E *** **−** **03	4.44*E *** **−** **05
	Std	7.09*E *** **−** **05	2.38*E *** **−** **04	2.68*E *** **−** **02	1.47*E *** **−** **02	**5.45E **−** 06**	6.79*E *** **−** **02	7.60*E *** **−** **02	5.30*E *** **−** **03	1.13*E *** **−** **04

F13	Mean	5.59*E *** **−** **02	7.47*E *** **−** **04	2.76*E* + 00	5.80*E* + 00	1.61*E *** **−** **04	6.80*E *** **−** **01	6.80*E* + 00	**1.15E **−** 04**	1.71*E *** **−** **03
	Std	2.09*E *** **−** **01	1.16*E *** **−** **03	1.01*E* + 00	8.37*E *** **−** **01	2.33*E *** **−** **04	2.45*E *** **−** **01	4.67*E *** **−** **01	**1.18E **−** 04**	3.99*E *** **−** **03

**Table 6:** The statistical results of Wilcoxon's rank-sum test (F1–F13).

Function	Dimension	EHO	WOA	EO	HHO	CSO	GWO	SFO	IEHO
F1	30	3.02*E *** **−** **11	3.02*E *** **−** **11	3.02*E *** **−** **11	3.02*E *** **−** **11	3.02*E *** **−** **11	3.02*E *** **−** **11	3.02*E *** **−** **11	3.02*E *** **−** **11
	50	3.02*E *** **−** **11	3.02*E *** **−** **11	3.02*E *** **−** **11	3.02*E *** **−** **11	3.02*E *** **−** **11	3.02*E *** **−** **11	3.02*E *** **−** **11	3.02*E *** **−** **11
	100	3.02*E *** **−** **11	3.02*E *** **−** **11	3.02*E *** **−** **11	3.02*E *** **−** **11	3.02*E *** **−** **11	3.02*E *** **−** **11	3.02*E *** **−** **11	3.02*E *** **−** **11

F2	30	3.02*E *** **−** **11	3.02*E *** **−** **11	3.02*E *** **−** **11	3.02*E *** **−** **11	3.02*E *** **−** **11	3.02*E *** **−** **11	3.02*E *** **−** **11	3.02*E *** **−** **11
	50	3.02*E *** **−** **11	3.02*E *** **−** **11	3.02*E *** **−** **11	3.02*E *** **−** **11	3.02*E *** **−** **11	3.02*E *** **−** **11	3.02*E *** **−** **11	3.02*E *** **−** **11
	100	3.02*E *** **−** **11	3.02*E *** **−** **11	3.02*E *** **−** **11	3.02*E *** **−** **11	3.02*E *** **−** **11	3.02*E *** **−** **11	3.02*E *** **−** **11	3.02*E *** **−** **11

F3	30	3.02*E *** **−** **11	3.02*E *** **−** **11	3.02*E *** **−** **11	3.02*E *** **−** **11	3.02*E *** **−** **11	3.02*E *** **−** **11	3.02*E *** **−** **11	3.02*E *** **−** **11
	50	3.01*E *** **−** **11	3.01*E *** **−** **11	3.01*E *** **−** **11	3.01*E *** **−** **11	3.01*E *** **−** **11	3.01*E *** **−** **11	3.01*E *** **−** **11	3.01*E *** **−** **11
	100	3.02*E *** **−** **11	3.02*E *** **−** **11	3.02*E *** **−** **11	3.02*E *** **−** **11	3.02*E *** **−** **11	3.02*E *** **−** **11	3.02*E *** **−** **11	3.02*E *** **−** **11

F4	30	3.02*E *** **−** **11	3.02*E *** **−** **11	3.02*E *** **−** **11	3.02*E *** **−** **11	3.02*E *** **−** **11	3.02*E *** **−** **11	3.02*E *** **−** **11	3.02*E *** **−** **11
	50	3.02*E *** **−** **11	3.02*E *** **−** **11	3.02*E *** **−** **11	3.02*E *** **−** **11	3.02*E *** **−** **11	3.02*E *** **−** **11	3.02*E *** **−** **11	3.02*E *** **−** **11
	100	3.02*E *** **−** **11	3.02*E *** **−** **11	3.02*E *** **−** **11	3.02*E *** **−** **11	3.02*E *** **−** **11	3.02*E *** **−** **11	3.02*E *** **−** **11	3.02*E *** **−** **11

F5	30	**9.63E **−** 02**	3.02*E *** **−** **11	3.02*E *** **−** **11	8.15*E *** **−** **05	6.07*E *** **−** **11	3.02*E *** **−** **11	1.00*E *** **−** **03	2.15*E *** **−** **02
	50	**9.00E **−** 01**	3.02*E *** **−** **11	3.02*E *** **−** **11	1.78*E *** **−** **04	3.34*E *** **−** **11	3.02*E *** **−** **11	**5.94E **−** 02**	**5.89E **−** 01**
	100	**4.83E **−** 01**	3.02*E *** **−** **11	3.02*E *** **−** **11	1.03*E *** **−** **02	3.02*E *** **−** **11	3.02*E *** **−** **11	**2.23E **−** 01**	**8.65E **−** 01**

F6	30	2.89*E *** **−** **03	5.61*E *** **−** **05	5.96*E *** **−** **09	6.35*E *** **−** **05	3.02*E *** **−** **11	1.63*E *** **−** **05	8.14*E *** **−** **05	5.32*E *** **−** **03
	50	9.79*E *** **−** **05	1.61*E *** **−** **06	**5.69E **−** 01**	3.96*E *** **−** **08	1.16*E *** **−** **07	1.11*E *** **−** **06	1.86*E *** **−** **03	1.68*E *** **−** **03
	100	6.28*E *** **−** **06	2.77*E *** **−** **05	4.94*E *** **−** **05	1.43*E *** **−** **08	7.20*E *** **−** **05	9.51*E *** **−** **06	1.61*E *** **−** **06	9.79*E *** **−** **05

F7	30	**9.59E **−** 01**	1.41*E *** **−** **04	1.75*E *** **−** **05	1.17*E *** **−** **05	2.83*E *** **−** **08	3.08*E *** **−** **08	**3.18E **−** 01**	**1.09E **−** 01**
	50	**1.05E **−** 01**	6.36*E *** **−** **05	7.20*E *** **−** **05	3.32*E *** **−** **06	4.98*E *** **−** **11	2.83*E *** **−** **08	**4.55E **−** 01**	1.68*E *** **−** **03
	100	1.70*E *** **−** **02	1.25*E *** **−** **04	2.20*E *** **−** **07	6.05*E *** **−** **07	3.02*E *** **−** **11	3.69*E *** **−** **11	**4.73E **−** 01**	**4.04E **−** 01**

F8	30	3.56*E *** **−** **04	4.98*E *** **−** **11	3.02*E *** **−** **11	1.68*E *** **−** **04	1.09*E *** **−** **10	3.02*E *** **−** **11	3.02*E *** **−** **11	2.60*E *** **−** **05
	50	**3.71E **−** 01**	2.87*E *** **−** **10	3.02*E *** **−** **11	**6.20E **−** 01**	3.02*E *** **−** **11	3.02*E *** **−** **11	3.02*E *** **−** **11	**2.64E **−** 01**
	100	3.56*E *** **−** **04	1.21*E *** **−** **10	3.02*E *** **−** **11	**9.00E **−** 01**	3.02*E *** **−** **11	3.02*E *** **−** **11	3.02*E *** **−** **11	3.67*E *** **−** **03

F9	30	1.21*E *** **−** **12	**8.15E **−** 02**	**3.34E **−** 01**	**NaN**	1.21*E *** **−** **12	1.20*E *** **−** **12	1.21*E *** **−** **12	1.21*E *** **−** **12
	50	1.21*E *** **−** **12	**3.34E **−** 01**	**3.34E **−** 01**	**NaN**	1.21*E *** **−** **12	1.21*E *** **−** **12	1.21*E *** **−** **12	1.21*E *** **−** **12
	100	1.21*E *** **−** **12	**NaN**	**NaN**	**NaN**	1.21*E *** **−** **12	1.21*E *** **−** **12	1.21*E *** **−** **12	1.21*E *** **−** **12

F10	30	1.21*E *** **−** **12	8.07*E *** **−** **08	6.12*E *** **−** **14	**NaN**	1.21*E *** **−** **12	1.16*E *** **−** **12	1.21*E *** **−** **12	1.21*E *** **−** **12
	50	1.21*E *** **−** **12	2.74*E *** **−** **09	2.59*E *** **−** **13	**NaN**	1.21*E *** **−** **12	1.21*E *** **−** **12	1.21*E *** **−** **12	1.21*E *** **−** **12
	100	1.21*E *** **−** **12	7.78*E *** **−** **10	7.78*E *** **−** **13	**NaN**	1.21*E *** **−** **12	1.21*E *** **−** **12	1.21*E *** **−** **12	1.21*E *** **−** **12

F11	30	1.21*E *** **−** **12	**3.34E **−** 01**	**NaN**	**NaN**	1.21*E *** **−** **12	5.58*E *** **−** **03	4.57*E *** **−** **12	1.21*E *** **−** **12
	50	1.21*E *** **−** **12	**3.34E **−** 01**	**NaN**	**NaN**	1.21*E *** **−** **12	3.13*E *** **−** **04	1.21*E *** **−** **12	1.21*E *** **−** **12
	100	1.21*E *** **−** **12	**NaN**	**3.34E **−** 01**	**NaN**	1.21*E *** **−** **12	1.21*E *** **−** **12	1.21*E *** **−** **12	1.21*E *** **−** **12

F12	30	**9.82E **−** 01**	4.50*E *** **−** **11	6.77*E *** **−** **05	**2.71E **−** 01**	3.02*E *** **−** **11	3.02*E *** **−** **11	**8.77E **−** 01**	8.07*E *** **−** **04
	50	**3.55E **−** 01**	3.02*E *** **−** **11	6.74*E *** **−** **06	**1.37E **−** 01**	4.64*E *** **−** **03	3.02*E *** **−** **11	**1.49E **−** 01**	9.12*E *** **−** **03
	100	**1.09E **−** 01**	3.02*E *** **−** **11	3.02*E *** **−** **11	1.52*E *** **−** **03	6.70*E *** **−** **11	3.02*E *** **−** **11	**2.12E **−** 01**	1.81*E *** **−** **04

F13	30	**3.87E **−** 01**	3.02*E *** **−** **11	**2.28E **−** 01**	**1.67E **−** 01**	3.02*E *** **−** **11	3.02*E *** **−** **11	**8.42E **−** 01**	**5.11E **−** 01**
	50	**9.00E **−** 01**	3.02*E *** **−** **11	4.50*E *** **−** **11	**2.12E **−** 01**	7.29*E *** **−** **03	3.02*E *** **−** **11	**3.33E **−** 01**	**1.02E **−** 01**
	100	**6.41E **−** 01**	3.02*E *** **−** **11	3.02*E *** **−** **11	2.42*E *** **−** **02	3.02*E *** **−** **11	3.02*E *** **−** **11	**9.05E **−** 02**	**8.42E **−** 01**

+/ = /−	30	9/0/4	11/0/2	10/1/2	8/3/2	13/0/0	13/0/0	10/0/3	11/0/2
	50	8/0/5	11/0/2/	10/1/2	7/3/3	13/0/0	13/0/0	9/0/4	10/0/3
	100	10/0/3	11/2/0	11/1/1	9/3/1	13/0/0	13/0/0	9/0/4	10/0/3

**Table 7:** The statistical results of Wilcoxon's rank-sum test (F14–F23).

Function	EHO	WOA	EO	HHO	CSO	GWO	SFO	IEHO
F14	5.57*E *** **−** **03	3.67*E *** **−** **03	1.01*E *** **−** **11	**8.77E **−** 01**	**1.61E **−** 01**	5.19*E *** **−** **07	3.02*E *** **−** **11	4.68*E *** **−** **02
F15	6.36*E *** **−** **05	4.62*E *** **−** **10	1.07*E *** **−** **07	3.02*E *** **−** **11	7.74*E *** **−** **06	1.11*E *** **−** **06	3.02*E *** **−** **11	**5.01E **−** 02**
F16	**2.97E **−** 01**	3.02*E *** **−** **11	1.14*E *** **−** **11	3.02*E *** **−** **11	1.69*E *** **−** **09	3.02*E *** **−** **11	1.73*E *** **−** **07	**6.63E **−** 01**
F17	2.07*E *** **−** **02	3.02*E *** **−** **11	1.21*E *** **−** **12	3.68*E *** **−** **11	1.01*E *** **−** **08	3.69*E *** **−** **11	1.31*E *** **−** **08	2.05*E *** **−** **03
F18	1.86*E *** **−** **03	3.02*E *** **−** **11	2.29*E *** **−** **11	3.02*E *** **−** **11	4.20*E *** **−** **10	5.57*E *** **−** **10	7.66*E *** **−** **05	3.18*E *** **−** **04
F19	1.08*E *** **−** **02	7.39*E *** **−** **11	6.32*E *** **−** **12	3.34*E *** **−** **11	1.17*E *** **−** **09	3.02*E *** **−** **11	1.86*E *** **−** **09	**7.73E **−** 02**
F20	**3.87E **−** 01**	3.02*E *** **−** **11	1.82*E *** **−** **11	3.34*E *** **−** **11	3.02*E *** **−** **11	3.02*E *** **−** **11	3.20*E *** **−** **09	9.82*E *** **−** **05
F21	2.81*E *** **−** **02	1.03*E *** **−** **06	**2.45E **−** 01**	3.02*E *** **−** **11	7.66*E *** **−** **03	**5.79E **−** 01**	4.62*E *** **−** **10	1.02*E *** **−** **05
F22	**4.12E **−** 01**	3.09*E *** **−** **06	5.75*E *** **−** **05	3.02*E *** **−** **11	7.96*E *** **−** **03	**6.31E **−** 01**	6.01*E *** **−** **08	**3.18E **−** 01**
F23	**1.71E **−** 01**	2.19*E *** **−** **08	2.83*E *** **−** **10	3.02*E *** **−** **11	6.77*E *** **−** **05	**4.12E **−** 01**	1.70*E *** **−** **08	1.08*E *** **−** **02
+/ = /−	6/0/4	10/0/0	9/0/1	9/0/1	9/0/1	7/0/0	10/0/0	6/0/4

**Table 8:** Results of Friedman test on 23 benchmark functions.

Function	Dimension		SRGS-EHO	EHO	WOA	EO	HHO	CSO	GWO	SFO	IEHO
F1–F13	30	Friedman value	2.462	4.682	5.218	4.231	5.769	6.769	5.615	5.231	5.077
		Friedman rank	1	3	5	2	8	9	7	6	4
	50	Friedman value	2.615	4.846	5.308	4.692	5.385	5.462	6.154	4.154	6.385
		Friedman rank	1	4	5	3	6	7	8	2	9
	100	Friedman value	2.279	4.154	6.538	5.149	4.615	6.154	4.308	5.846	5.923
		Friedman rank	1	2	9	5	4	8	3	6	7

F14–F23	Fixed	Friedman value	1.925	3.731	5.975	6.626	5.737	6.442	3.858	5.622	5.404
		Friedman rank	1	2	7	9	6	8	3	5	4

**Table 9:** Combination of different parameters in SRGS-EHO.

Parameters		SRGS-EHO1	SRGS-EHO2	SRGS-EHO3	SRGS-EHO4	SRGS-EHO5	SRGS-EHO6	SRGS-EHO7	SRGS-EHO8	SRGS-EHO9	SRGS-EHO10	SRGS-EHO11	SRGS-EHO12
*t*_max_	100	√	√	√	√	√	√						
	500							√	√	√	√	√	√

*N*	5	√			√			√			√		
	20		√			√			√			√	
	50			√			√			√			√

*a*, *b*	*a* = −*π*												
	*b* = *π*	√	√	√				√	√	√			
	*a* = 0												
	*b* = 1			√	√	√				√	√	√	

**Table 10:** Comparison results by Friedman test for different versions of SRGS-EHO on 23 benchmark functions.

Functions	SRGS-EHO1	SRGS-EHO2	SRGS-EHO3	SRGS-EHO4	SRGS-EHO5	SRGS-EHO6	SRGS-EHO7	SRGS-EHO8	SRGS-EHO9	SRGS-EHO10	SRGS-EHO11	SRGS-EHO12
F1	9.6000	3.2667	9.0667	3.5333	9.1333	3.4000	9.6333	3.4000	9.8000	3.8667	9.7667	3.5333
F2	9.2000	3.5667	9.3333	3.3333	9.6667	2.7667	9.6000	3.6333	9.4000	3.8667	9.8000	3.8333
F3	9.9667	3.2667	9.8000	3.5000	9.4000	3.7333	9.1000	3.4000	9.0333	3.4000	9.7000	3.7000
F4	9.4000	3.2000	9.7000	3.3333	9.6000	3.6667	9.0333	3.5333	9.2333	3.3667	10.0333	3.9000
F5	8.3333	6.3333	7.9667	4.7333	8.8000	3.4667	9.2667	5.1667	7.1333	5.2000	7.9667	3.6333
F6	7.5000	5.9000	8.5000	3.9333	7.6000	4.0333	8.2667	4.8667	8.5000	4.8000	9.1667	4.9333
F7	9.5333	5.8000	8.0000	4.3000	7.5000	3.5667	9.2000	5.7667	8.8000	4.1333	8.2333	3.1667
F8	8.8000	4.6333	7.3667	4.8000	8.9000	4.6667	8.2667	4.9000	8.7333	4.0667	8.9000	3.9667
F9	1.0000	1.0000	1.0000	1.0000	1.0000	1.0000	1.0000	1.0000	1.0000	1.0000	1.0000	1.0000
F10	1.0000	1.0000	1.0000	1.0000	1.0000	1.0000	1.0000	1.0000	1.0000	1.0000	1.0000	1.0000
F11	1.0000	1.0000	1.0000	1.0000	1.0000	1.0000	1.0000	1.0000	1.0000	1.0000	1.0000	1.0000
F12	9.4000	4.9333	7.9667	3.7333	8.3000	3.6000	9.1667	5.2000	8.6000	4.8000	8.8333	3.4667
F13	8.6000	5.5667	8.7667	4.4000	7.5667	3.0667	8.5333	5.6000	9.4333	4.4000	8.3333	3.7333
F14	4.7333	6.8333	5.4333	7.2333	6.5333	7.5000	5.6000	6.0000	7.7333	7.0333	6.5333	6.8333
F15	8.6667	5.4333	8.5333	4.2667	8.4000	4.2333	7.5667	5.0667	8.9000	4.4000	7.7333	4.8000
F16	8.2000	8.8667	6.6333	4.4000	5.4000	4.5000	9.0667	8.9000	8.0667	4.8333	5.1333	4.0000
F17	8.8000	5.9667	9.4000	5.1667	6.3000	4.3667	8.6333	5.7667	7.2000	4.6667	7.4667	4.2667
F18	9.2000	8.2000	6.2333	5.5667	4.2667	4.5333	9.6667	8.3667	6.8333	6.5000	4.0667	4.5667
F19	10.4333	8.8667	6.0333	5.4000	4.3667	3.7333	8.6000	9.5333	6.1000	6.4667	3.7667	4.7000
F20	9.4667	8.6667	7.5000	6.0000	3.6000	4.7333	9.2000	8.6333	6.0667	6.4333	3.3667	4.3333
F21	8.2000	4.6000	7.8333	4.5333	8.5333	4.7333	9.4667	5.4000	7.2333	4.7000	8.9000	3.8667
F22	8.0333	5.4000	8.1667	4.9000	7.2333	4.3000	9.4000	5.3667	8.2667	4.4667	8.7000	3.7667
F23	8.7667	4.9000	8.2000	4.7667	9.1333	3.7667	8.4000	4.6000	7.7333	4.3667	8.9667	4.4000
Average rank	7.7319	5.0957	7.1058	4.1232	6.6623	3.7116	7.7681	5.0478	7.2087	4.2942	6.8855	3.7565
Overall rank	11	6	9	3	7	1	12	5	10	4	8	2

**Table 11:** Combination of different parameters in SRGS-EHO.

	SR-GM	GSO
EHO	0	0
SR-GM + EHO	1	0
GSO + EHO	0	1
SRGS-EHO	1	1

**Table 12:** Comparison results for different combinations on 6 benchmark functions.

Functions	EHO	SR-GM + EHO	GSO + EHO	SRGS-EHO
F1	3.54*E* − 05	4.99*E* − 07	4.73*E* − 277	**3.60E** − **313**
F5	1.03*E* − 01	1.99*E* − 02	2.71*E* − 02	**3.32E** − **03**
F10	7.08*E* − 04	1.22*E* − 03	**8.88E** − **16**	**8.88E** − **16**
F14	9.98*E* − 01	9.98*E* − 01	9.98*E* − 01	**9.99E** − **01**
F15	1.67*E* − 03	**1.67E** − **03**	1.68*E* − 03	1.67*E* − 03
F17	4.18*E* − 01	3.99*E* − 01	3.99*E* − 01	**3.98E** − **01**
Average rank	2.8536	2.8	2.1444	1.7852
Overall rank	4	3	2	1

**Table 13:** Comparison results of pressure-vessel design problem.

Algorithm	Optimal values for variables				Optimum cost
	*T*_*s*_	*T*_*h*_	*R*	*L*	
SRGS-EHO	0.850468	0.420387	44.065679	153.694517	6020.753071
EO	0.898401	0.444080	46.549292	128.317630	6124.239342
WOA	1.040632	0.511766	50.905188	91.322007	6775.807533
HHO	1.079160	0.543392	55.469516	60.115203	6715.912450
DE	0.812500	0.437500	42.098353	176.637751	6059.725800
ES	0.812500	0.437500	42.098087	176.640518	6059.745600
PSO	0.812500	0.437500	42.091266	176.746500	6061.077700
OBSCA	3.000000	0.875000	66.148100	159.303600	6958.988200
ISCA	0.8125	0.4375	42.09842	176.6382	6059.745738
EWOA	10.0625	0.50	58.17399	44.38294	6177.754912

**Table 14:** Comparison results of the problem of tension/compression spring design.

Algorithms	Optimal values for variables			Optimum weight
	*d*	*D*	*N*	
SRGS-EHO	0.061414	0.638027	3.004913	0.012044
SSA	0.051207	0.345215	12.004032	0.012676
WOA	0.053234	0.395036	9.351476	0.012708
PSO	0.015728	0.357644	11.244543	0.012675
GA	0.051480	0.351661	11.632201	0.012705
MFO	0.051994	0.364109	10.868422	0.012667
GWO	0.051690	0.356760	11.288110	0.012662
EWOA	0.051961	0.363306	10.91296	0.012667
EHOI	0.051594	0.354438	11.423880	0.012665
RDWOA	0.0517112	0.35725	11.257788	0.012665

## Data Availability

The data used to support the findings of this study are available from https://github.com/dyxdddddd/SRGS-EHO.
